# An Embedded Multiscale Modelling to Guide Control and Elimination of Paratuberculosis in Ruminants

**DOI:** 10.1155/2021/9919700

**Published:** 2021-11-26

**Authors:** Rendani Netshikweta, Winston Garira

**Affiliations:** Modelling Health and Environmental Linkages Research Group (MHELRG), Department of Mathematics and Applied Mathematics, University of Venda, Private Bag X5050, Thohoyandou 0950, South Africa

## Abstract

In recent years, multiscale modelling approach has begun to receive an overwhelming appreciation as an appropriate technique to characterize the complexity of infectious disease systems. In this study, we develop an embedded multiscale model of paratuberculosis in ruminants at host level that integrates the within-host scale and the between-host. A key feature of embedded multiscale models developed at host level of organization of an infectious disease system is that the within-host scale and the between-host scale influence each other in a reciprocal (i.e., both) way through superinfection, that is, through repeated infection before the host recovers from the initial infectious episode. This key feature is demonstrated in this study through a multiscale model of paratuberculosis in ruminants. The results of this study, through numerical analysis of the multiscale model, show that superinfection influences the dynamics of paratuberculosis only at the start of the infection, while the MAP bacteria replication continuously influences paratuberculosis dynamics throughout the infection until the host recovers from the initial infectious episode. This is largely because the replication of MAP bacteria at the within-host scale sustains the dynamics of paratuberculosis at this scale domain. We further use the embedded multiscale model developed in this study to evaluate the comparative effectiveness of paratuberculosis health interventions that influence the disease dynamics at different scales from efficacy data.

## 1. Introduction

In the field of mathematical biology, we are beginning to witness an overwhelming appreciation of multiscale modelling in studying infectious disease systems dynamics (see [1–7] and references therein). The complexity of an infectious disease system arises from the interactions of three main subsystems which are the host subsystem, the pathogen subsystem, and the environment subsystem [8]. It is worthy noting that the foundations for development of multiscale models of infectious disease systems have been established in four main pivotal publications [7–10]. These publications introduced critical concepts and summarized them in a form that transformed mainstream thinking about the multiscale dynamics of infectious disease systems. The multiscale dynamics of infectious disease systems comes from the fact that pathogens select habitat at different hierarchical levels and at multiple scales (in space and time) within each hierarchical level. One of the foundational ideas established in [7, 8] is that infectious disease systems are organized into seven main levels of organization which are [7, 8] the cell level, the tissue level, the organ or microcommunity level, the microecosystem level, the host level, the macrocommunity level, and the macroecosystem level. For more details on the seven-level hierarchical framework of organization of an infectious disease system, see the key publications [7, 9, 10]. In the context of this seven-level hierarchical framework of organization of an infectious disease system, these publications established the fundamental idea that disease processes interact across scales in space and time, such that as the spatial scale of the phenomenon increases so does the temporal scale over which it operates. Another monumental contribution to the modern perspective on multiscale dynamics of infectious disease systems is that the multiscale modelling of infectious disease systems can be described by five main different categories of multiscale models which are [9, 10] (i) individual-based multiscale models (IMSMs), (ii) nested multiscale models (NMSMs), (iii) embedded multiscale models (EMSMs), (iv) hybrid multiscale models (HMSMs), and (v) coupled multiscale models (CMSMs). These five different categories of multiscale models of infectious disease systems can be developed at any of the seven main hierarchical levels of organization of an infectious disease system. However, in this study, we develop an embedded multiscale model that integrates two adjacent scales at the host level of organization (i.e., the within-host scale and the between-host scale) to investigate the influence of superinfection on the dynamics of infectious disease systems with a pathogen replication-cycle at the microscale using paratuberculosis as a paradigm.

A defining feature of embedded multiscale models is that at any level of organization of a disease system the macroscale influences the microscale through superinfection, that is, repeated infection before the host recovers from the initial infectious episode [7, 8]. This is unlike the nested multiscale models in which the macroscale influences the microscale through initial infective inoculum [7]. Thus, the main objective of this study is to investigate using an embedded multiscale model how superinfection influences disease dynamics for an infection with a pathogen replication-cycle at the microscale and further use the model to evaluate the comparative effectiveness of the health interventions that operate at different scale domains (i.e., the within-host scale and the between-host scale) of an infectious disease system using paratuberculosis in ruminants as a case study. To the best of our knowledge, there is no embedded multiscale model in the literature that we are aware of which characterizes the multiscale dynamics of an infectious disease that has a pathogen replication-cycle at the microscale of any of the 7 levels of organization of an infectious disease system [8]. The embedded multiscale model presented in this study is the first of its kind to be developed to characterize infectious disease dynamics with a pathogen replication-cycle at the microscale. However, the only embedded multiscale models that we aware of are for infectious disease systems without a pathogen replication-cycle at the microscale [1, 2, 4, 7].

Unlike infectious disease systems such as hookworm infection, Guinea worm infection and human schistosomiasis [2, 4, 7] in which their disease-causing agents have no replication-cycle at the microscale (i.e., within-host scale), paratuberculosis (PTB) in ruminants considered in this study as a paradigm is caused by a bacteria that has a replication-cycle at within-host scale. The bacteria which is responsible for PTB infection in ruminants is called *Mycobacterium Avium Subspecies Paratuberculosis* (MAP) [11–13]. This is one of the most notorious obligate pathogen affecting domestic ruminants and wild animals throughout the world [14–16]. MAP is commonly widespread in dairy cattle and can significantly pose serious economic burdens in dairy cattle industries due to the reduction of milk production, increased cattle mortality, and premature culling of infected cattle as well as reduction of sale price for cattle in regions with high PTB prevalence [17]. Moreover, clinical outcomes of PTB infection in ruminants such as dairy cattle is manifested through ruminant growth failure, increases in weight loss, and chronic diarrhea [15, 18]. The dynamics of PTB disease causing-bacteria (MAP bacteria) in the ruminant population involves the transmission of bacteria at between-host scale which usually occurs through a fecal-oral route [14]. It also involves the replication of the bacteria within an infected ruminant macrophages and the survival of the bacteria outside the ruminant host. For more details on the transmission, replication, and survival of MAP bacteria in ruminant populations, see the published works in [18, 19]. Here, we only provide a brief description. The transmission and replication processes of MAP bacteria in ruminant populations begin when a ruminant ingests fecal materials in the environment contaminated with MAP bacteria. After the ingestion, MAP bacteria reaches the intestines of the ruminant and is taken up by either M cells or enterocytes in the Peyers patches of the lower small intestine and transported to submucosal macrophages and then engulfed. At this stage of infection, some of the MAP bacteria will be destroyed by macrophages, and some will survive and replicate inside those macrophages. After some period, macrophages with replicating MAP bacteria burst to release the bacteria into the extracellular environment of the ruminant at the site of infection. At the later stage of infection, the ruminant begins to shed bacteria via feces into the environment. Then, the ingestion of the bacteria in the environment by other ruminant closes the replication-transmission multiscale cycle of PTB. However, the replication-transmission multiscale cycle of MAP bacteria can be interrupted by different health interventions that can be administrated either at within-host scale or at between-host scale. Currently, there is no drug that has been made available to combat the bacteria at within-host scale. The only control measures against the disease include (i) vaccination which is administrated at the within-host scale of the ruminant to increase resistance of ruminants to infection, (ii) environmental hygiene-management which is administrated at the between-host scale of ruminants to kill the MAP bacteria in the environment, and (iii) test and culling which is administrated at the between-host scale of the ruminant population to eliminate the sources of PTB infection in the herd. But all these control measures have limited success against PTB infection. For more details about the aforementioned health intervention measures and their limited success against PTB infection in ruminants, see [20].

In the past, multiscale modelling of PTB in ruminants at host level has been done. This involved the development of individual-based multiscale models (IMSMs) such as [21] and hybrid multiscale models (HMSMs) such as [13, 22]. It is also worth mentioning that although both IMSMs and HMSMs in [13, 21] have, respectively, shed some light into the multiscale nature of PTB infection and the impact of health interventions against this disease, there are important limitations of these categories of multiscale when compared with the embedded multiscale model presented in this study. The IMSMs cannot be easily used to evaluate the comparative effectiveness of health interventions using the often used disease transmission metrics such as reproductive numbers and endemic equilibria because it is not easy to derive explicit expressions of such quantities from these IMSMs. Similarly, HMSMs cannot also be easily applied to evaluate the comparative effectiveness of health interventions that operate at different scale domains such as within-host scale and between-host scale because they do not often use a common metric of disease transmission across scales. In addition, the majority of mathematical models for PTB infection are single-scale models (see [11, 12, 23–27] and references therein). We also note from the work in [10] that at any level of organization of an infectious disease systems of an organization (be cell-level, tissue-level, host-level, etc.), multiscale models can be more advantageous than single-scale-based models largely because multiscale models can be used to concurrently evaluate the effectiveness of health interventions that operate at different scales in the replication-transmission multiscale cycle of an infectious disease system. Single-scale-based models restrict themselves only to one part of the replication-transmission multiscale multiscale cycle of an infectious disease system.

The remainder of this paper is organized as follows. In Section 2, we present a baseline embedded multiscale model for PTB infection in ruminants. Mathematical analysis of this baseline embedded multiscale model is done in Section 3. In Section 4, this baseline embedded multiscale model is analyzed numerically to confirm some of the analytical results obtained in Section 3. In Section 5, we extend the baseline embedded multiscale in Section 2 to incorporate PTB health interventions and use it to evaluate the comparative effectiveness of the PTB health interventions. The paper ends with conclusions in Section 6.

## 2. Multiscale Model for Paratuberculosis Multiscale Cycle Dynamics in Ruminants

In order to explicitly characterize the replication-transmission multiscale cycle of PTB in ruminants and further ascertain the influence of superinfection on the dynamics of the disease, we develop a multiscale model which takes into account the reciprocal influences between the within-host scale (pathogen-cell interaction and replication) dynamics and between-host scale (circulation of pathogen in the host population) dynamics. Moreover, the replication-transmission multiscale cycle for PTB considered in this article is a primary multiscale cycle. For details of multiscale cycles in disease dynamics which include primary multiscale cycle, secondary multiscale cycle, and tertiary multiscale cycle, see the published works [7, 8, 10]. In the formulation of the embedded multiscale model for PTB dynamics, the PTB within-host scale submodel was adopted with minor modifications from a single-scale model framework in Magombedze et al. [12]. However, the only minor extension to the model in [12] is the addition of a parameter for excretion/shedding rate *α*_*c*_ of MAP into extracellular environment which is crucial for linking the two main disease processes of PTB which are the within-host scale pathogen replication and the between-host scale pathogen transmission. While the between-host submodel is based on a susceptible-infected-susceptible (SIS) epidemic framework. Integrating the between-host scale submodel and the adopted within-host scale submodel results in the proposed embedded multiscale model for ruminant paratuberculosis transmission-replication multiscale cycle which is consequently based on monitoring the dynamics of nine populations: susceptible ruminants (*S*_*C*_), infected ruminants (*I*_*C*_), and the MAP bacilli bacterial load (*B*_*C*_) in the environment at the between-host scale in the host population; susceptible macrophages (*M*_*Φ*_), infected macrophages (*I*_*m*_), and within-host MAP bacilli bacterial load (*B*_*c*_) at the within-host scale; and specific naive CD4+ T cells (*T*_0_), Th1 response cells (*T*_1_), and Th2 phenotype response cells (*T*_2_) at the within-host scale in the infected ruminant-host population. We make the following assumptions for this model:

- Infected ruminants can recover naturally from MAP infection
- Transmission of infection is only through indirect means, and if there is any direct transmission, it will be estimated by an indirect (environmental transmission) expression
- There is no vertical transmission, and ruminant hosts are not vaccinated or treated and so the infection state of the ruminant hosts (exposed, subclinical, clinical, etc.) is only determined by the within-host scale MAP dynamics
- The recruitment of ruminants in the herd is through birth and incoming ruminants from other farms
- All the new recruited ruminants are assumed to be healthy and have not been previously exposed to the disease
- The extracellular MAP bacterial load *B*_*c*_ = *B*_*c*_(*t*) is a proxy for individual ruminant infectiousness and is excreted out of the body of an individual ruminant through feces
- The depletion of MAP bacteria in the extracellular environment through engulfment by macrophages is negligible
- There is no bacteria replication in the physical environment, and the loss of MAP bacteria in the environment due to uptake of the parasite by susceptible ruminant hosts is negligible
- Clonal expansion of the *T*_0_ cells into *T*_1_ is only due to infected macrophages while clonal expansion of the *T*_2_ is only due to MAP bacteria in the infected ruminant host

Based on these assumptions, the embedded multiscale model for PTB transmission dynamics is governed by the following system of ordinary differential equations.

(1) $$\begin{array}{c} \left\{\begin{array}{cc} 1. & \frac{dS_{C}\left(t\right)}{dt}=\Lambda_{C}-\frac{\beta_{C}B_{C}\left(t\right)S_{C}\left(t\right)}{B_{0}+B_{C}\left(t\right)}-\mu_{C}S_{C}\left(t\right)+\gamma_{C}I_{C}\left(t\right),\\ 2. & \frac{dI_{C}\left(t\right)}{dt}=\frac{\beta_{C}B_{C}\left(t\right)S_{C}\left(t\right)}{B_{0}+B_{C}\left(t\right)}-\left[\mu_{C}+\delta_{C}+\gamma_{C}\right]I_{C}\left(t\right),\\ 3. & \frac{dB_{C}\left(t\right)}{dt}=\alpha_{c}\left[I_{C}\left(t\right)+1\right]B_{c}\left(t\right)-\alpha_{C}B_{C}\left(t\right),\\ 4. & \frac{dB_{c}\left(t\right)}{dt}=\frac{\beta_{C}B_{C}\left(t\right)\left[S_{C}\left(t\right)-1\right]}{\left[B_{0}+B_{C}\left(t\right)\right]\Phi_{C}\left[I_{C}\left(t\right)+1\right]}+N_{m}k_{m}I_{m}\left(t\right)-\left[\mu_{c}+\alpha_{c}\right]B_{c}\left(t\right),\\ 5. & \frac{dM_{\phi }\left(t\right)}{dt}=\Lambda_{\phi }-\beta_{\phi }M_{\phi }\left(t\right)B_{c}\left(t\right)-\mu_{\phi }M_{\phi }\left(t\right),\\ 6. & \frac{dI_{m}\left(t\right)}{dt}=\beta_{\phi }M_{\phi }\left(t\right)B_{c}\left(t\right)-\left[k_{m}+\mu_{\phi }\right]I_{m}\left(t\right)-\gamma_{m}T_{1}\left(t\right)I_{m}\left(t\right),\\ 7. & \frac{dT_{0}\left(t\right)}{dt}=\Lambda_{0}-\left[\delta_{m}I_{m}\left(t\right)+\delta_{b}B_{c}\left(t\right)\right]T_{0}\left(t\right)-\mu_{0}T_{0}\left(t\right),\\ 8. & \frac{dT_{1}\left(t\right)}{dt}=\theta_{1}\delta_{m}I_{m}\left(t\right)T_{0}\left(t\right)-\mu_{1}T_{1}\left(t\right),\\ 9. & \frac{dT_{2}\left(t\right)}{dt}=\theta_{2}\delta_{b}B_{c}\left(t\right)T_{0}\left(t\right)-\mu_{2}T_{2}\left(t\right). \end{array}\right. \end{array}$$

Further, the embedded multiscale model (1) is schematically represented by Figure 1. In this PTB embedded multiscale model, the two submodels (within-host scale submodel and between-host scale submodel) are linked through a method well established in [1, 2, 4, 7]. In the first two equations of the multiscale model system (1), equations (1) and (2) describe the dynamics of susceptible and infected ruminant hosts, respectively. At any time *t*, new recruits of susceptible ruminants enter the ruminant population through birth and incoming ruminants from other farms at a constant rate *Λ*_*C*_. Susceptible ruminant population losses its individuals due to natural death at a constant rate *μ*_*C*_ and through infection at a variable rate *β*_*C*_*B*_*C*_(*t*)*S*_*C*_(*t*)/(*B*_0_ + *B*_*C*_(*t*)). We also assume that the population of susceptible ruminants increases through recovery of infected individuals at a rate *γ*_*C*_. Susceptible ruminants acquire PTB infection when they feed from contaminated pasture with fecal material containing infective MAP or drink from contaminated surface water/water troughs with MAP bacilli cells. The infected ruminants are generated when susceptible ruminants become infected and join the group at a rate variable *β*_*C*_*B*_*C*_(*t*)*S*_*C*_(*t*)/(*B*_0_ + *B*_*C*_(*t*)). The infected group decreases due to natural death at a constant rate *μ*_*C*_ or through disease induced death at rate *δ*_*C*_ or through recovery at a rate *γ*_*C*_ so that an average lifespan of PTB infected ruminant in the population is determined by 1/(*δ*_*C*_ + *μ*_*C*_ + *γ*_*C*_). Following the method in [1, 2, 4, 7], we assume that infected ruminants spread the disease in the population through contaminating the environment with fecal material containing the MAP bacteria cells at a variable rate *α*_*c*_*B*_*c*_(*t*)(*I*_*C*_(*t*) + 1) as shown in Figure 1. Therefore, the population dynamics of MAP bacilli in the physical environment, described by equation (3) of the model system (1), is generated through excretion/shedding of fecal material containing the MAP bacteria cells by infected ruminant host at a variable rate *α*_*c*_*B*_*c*_(*t*)(*I*_*C*_(*t*) + 1). Further, we also assume that the population of MAP bacteria in the physical environment decreases due to natural death at a rate *α*_*C*_. Equation (4) of the model system (1) describes the changes in time of the within-host MAP bacteria cells at the site of infection within a single infected ruminant host. The within-host MAP bacteria cells at the site of infection within an infected ruminant host are generated following uptake of average between-host MAP bacteria cells in the physical environment through ingesting of contaminated food or water and the release of the intracellular MAP bacilli into the extracellular environment when each infected macrophage bursts. In general, in the ruminant population, the uptake of contaminated food or water, which contains between-host MAP bacterial cells, is the transmission of the MAP bacteria from the physical environment to susceptible ruminant and become infected ruminant. Following the methodology described in [2, 4] for modelling superinfection for environmentally transmitted infectious disease systems, we model the average rate at which a single susceptible ruminant host uptake MAP bacteria cells in the physical environment through ingesting contaminated food or water and become an infected ruminant host by the expression

(2) $$\begin{array}{c} \lambda_{c}\left(t\right)S_{c}\left(t\right)=\frac{\beta_{C}B_{C}\left(t\right)S_{C}\left(\text{t}\right)}{B_{0}+B_{C}\left(t\right)}.\frac{\left[S_{C}\left(t\right)-1\right]}{\Phi_{C}\left[I_{C}\left(t\right)+1\right]}, \end{array}$$

so that the infection of a single host is defined by [4]:

(3) $$\begin{array}{c} \;\left(S_{C}\left(t\right),I_{C}\left(t\right),B_{C}\left(t\right)\right)⟶\left(S_{C}\left(t\right)-1,I_{C}\left(t\right)+1,B_{C}\left(t\right)\right). \end{array}$$

At the within-host scale PTB dynamics, infected macrophages burst at constant rate *k*_*m*_ to release an average number of intracellular MAP bacilli *N*_*m*_ into the extracellular environment, so that the total number of intracellular bacteria released into the extracellular environment is given by *N*_*m*_*k*_*m*_*I*_*m*_. Therefore, the average number of within-host MAP bacteria cells at the site of infection within an infected ruminant *B*_*c*_(*t*) within a single infected ruminant host increases at a mean rate *λ*_*h*_(*t*)*S*_*h*_(*t*) and *N*_*m*_*k*_*m*_*I*_*m*_. We assume that the population of MAP bacilli in the extracellular environment decay naturally at a constant rate *μ*_*c*_ and excreted out of the body of an infected ruminant into the physical environment through fecal material at a constant rate *α*_*c*_. Equations (5) and (6) of the model system (1) describe the dynamics of the susceptible macrophage cells *M*_*ϕ*_(*t*) and infected macrophage cells *I*_*m*_(*t*) at the site of infection within a single infected ruminant host. Similarly, at any time *t*, new susceptible macrophages are recruited through the supply of macrophage cells from progenitor monocytes that are recruited from the blood to the site of infection at a constant rate *Λ*_*ϕ*_, and the population losses individuals due to natural death at a constant rate *μ*_*ϕ*_. Susceptible macrophages acquire infection through engulfing extracellular MAP bacilli bacteria at a rate *β*_*ϕ*_. The infected macrophage cells at the site of infection within an infected ruminant host are generated when susceptible macrophages become infected and join the group of infected macrophages at a rate *β*_*ϕ*_. We assume that in the population of infected macrophages there is an additional death related to infection and due to removal by CD4 T ^+^ response cells at a rate *k*_*m*_ and *γ*_*m*_, respectively, so that the lifespan in the population of infected macrophages is 1/(*k*_*m*_ + *μ*_*ϕ*_ + *γ*_*m*_*T*_1_). The last three equations of the model system (1), equations (7)–(9), describe the evolution in time of the population of ruminant immune response cells at a site of infection in the gut which are specific naive CD4 T ^+^ cells (*T*_0_) and the two subsets of the MAP specific immune response, Th1 (*T*_1_) and Th2 (*T*_2_) cells (see [12] and reference therein). The population of specific naive CD4 T ^+^ cells (*T*_0_) for MAP bacilli are produced at a constant rate *Λ*_0_ from the thymus. We assume that these naive CD4 T ^+^ cells decay naturally at a rate *μ*_0_, so that their average lifespan is 1/*μ*_0_. Following the work in [12], we also assume that *T*_0_ cells become *T*_1_ and *T*_2_ immune response cells at per capita rates *δ*_*m*_ and *δ*_*b*_, respectively. Thus, the population of *T*_1_ and *T*_2_ immune response cells are proliferated at a rate *θ*_1_*δ*_*m*_*I*_*m*_*T*_0_ and *θ*_1_*δ*_*b*_*B*_*m*_*T*_0_, respectively. We further assume that both the population of *T*_1_ and *T*_2_ immune response cells decay naturally at a rate *μ*_1_ and *μ*_2_, respectively.

Figure 1 is a conceptual representation of the embedded multiscale model (1). The description of the PTB embedded multiscale model (1) and its parameter values used for model simulations are tabulated in Tables 1 and 2, respectively.

## 3. Mathematical Analysis of the Multiscale Model for Ruminant PTB Multiscale Cycle Dynamics

In this section, we present some mathematical analysis results of the PTB embedded multiscale model system (1). Mathematical analysis of the properties for the PTB embedded multiscale model system (1) is conducted in the region Γ ∈ *R*_+_^9^ of biological interest, which is given by:

(4) $$\begin{array}{c} \left\{\Gamma =\left\{\left(S_{C},I_{C},B_{C},B_{c},M_{\phi },I_{m},T_{0},T_{1},T_{2}\right)\in R_{+}^{9}:0\leq S_{C}+I_{C}\leq S_{1},0\leq M_{\phi }+I_{m}\leq S_{2},0\leq B_{C}\leq S_{3},0\leq B_{c}\leq S_{4},0\leq T_{0}\leq S_{5},0\leq T_{1}\leq S_{6},0\leq T_{2}\leq S_{7}\right\},\right. \end{array}$$

where

(5) $$\begin{array}{c} \left\{\begin{array}{c} S_{1}=\frac{\Lambda_{C}}{\mu_{C}},S_{2}=\frac{\Lambda_{\phi }}{\mu_{\phi }},S_{3}=\frac{\alpha_{c}\left(\Lambda_{C}+\mu_{C}\right)}{2\mu_{C}\alpha_{C}}\left[\xi_{1}+\sqrt{\xi_{1}^{2}+4\xi_{2}}\right],\\ S_{4}=\frac{1}{2}\left[\xi_{1}+\sqrt{\xi_{1}^{2}+4\xi_{2}}\right],S_{5}=\frac{\Lambda_{0}}{\mu_{0}},S_{6}=\frac{\theta_{1}\delta_{m}\Lambda_{0}\Lambda_{\phi }}{\mu_{\phi }\mu_{1}\mu_{0}},\\ S_{7}=\frac{\theta_{2}\delta_{b}\Lambda_{0}}{2\mu_{0}\mu_{2}}\left[\xi_{1}+\sqrt{\xi_{1}^{2}+4\xi_{2}}\right],\xi_{1}=\nu_{0}\left(\nu_{1}+\nu_{2}\right)-B_{0},\xi_{2}=\nu_{0}\nu_{2}B_{0},\\ \nu_{0}=\frac{\alpha_{c}\left(\Lambda_{C}+\mu_{C}\right)}{\mu_{C}\alpha_{C}},\nu_{1}=\frac{\beta_{C}\left(\Lambda_{C}-\mu_{C}\right)}{\Phi_{C}\left(\Lambda_{C}+\mu_{C}\right)\left(\mu_{c}+\alpha_{c}\right)},\nu_{2}=\frac{N_{m}k_{m}\Lambda_{\phi }}{\mu_{\phi }\left(\mu_{c}+\alpha_{c}\right)}. \end{array}\right. \end{array}$$

It can be easily shown that all solutions for the PTB embedded multiscale model system (1) with nonnegative initial conditions remain bounded within the invariant region Γ given by (4). Therefore, we conclude that the PTB embedded multiscale model system (1) is mathematically and epidemiologically well-posed [28]. Hence, it is sufficient to consider the dynamics of the flow generated by the PTB embedded multiscale model system (1) in Γ whenever *Λ*_*C*_ > *μ*_*C*_ and *ν*_0_(*ν*_1_ + *ν*_2_) > *B*_0_. We assume in all that follows (unless stated otherwise) that *Λ*_*C*_ > *μ*_*C*_ and *ν*_0_(*ν*_1_ + *ν*_2_) > *B*_0_. Details of the feasibility of the region Γ ∈ *R*_+_^9^ are given in Appendix A. In the next three subsections, we provide some results concerning the equilibrium states (i.e., the disease-free equilibrium state and the endemic equilibrium state) of the PTB embedded multiscale model system (1) and their stabilities.

### 3.1. The Disease-Free Equilibrium and Reproductive Number

We obtain the disease-free equilibrium point (DEF) of the PTB embedded multiscale model system (1) by setting the left-hand side of the equations of PTB multiscale model system (1) equal to zero and also assume that *I*_*C*_ = *B*_*C*_ = *B*_*c*_ = *I*_*m*_ = *T*_1_ = *T*_2_ = 0. Thus,

(6) $$\begin{array}{c} E_{0}=\left(\frac{\Lambda_{C}}{\mu_{C}},0,0,0,\frac{\Lambda_{\phi }}{\mu_{\phi }},0,\frac{\Lambda_{0}}{\mu_{0}},0,0\right), \end{array}$$

denotes the disease-free equilibrium of the PTB multiscale model system (1). For the purpose of analyzing the stability of the DFE, we make use of the basic reproduction number *R*_0_. The basic reproduction number of the system model (1) is calculated in this section using next generation operator approach described in [29]. Thus, the PTB multiscale model model system (1) can also be written in the form

(7) $$\begin{array}{c} \left\{\begin{array}{c} \frac{dX}{dt}=f\left(X,Y,Z\right),\\ \frac{dY}{dt}=g\left(X,Y,Z\right),\\ \frac{dZ}{dt}=h\left(X,Y,Z\right), \end{array}\right. \end{array}$$

where

- *X* = (*S*_*C*_, *M*_*ϕ*_, *T*_0_, *T*_1_, *T*_2_) represents all compartments of individuals who are not infected
- *Y* = (*I*_*C*_, *I*_*m*_) represents all compartments of infected individuals who are not capable of infecting others
- *Z* = (*B*_*C*_, *B*_*c*_) represents all compartments of infected individuals who are capable of infecting

In this case, we let the disease free-equilibrium of the model (1) be denoted by the following expression

(8) $$\begin{array}{c} {\bar{U}}_{0}=\left(\frac{\Lambda_{C}}{\mu_{C}},0,0,0,\frac{\Lambda_{\phi }}{\mu_{\phi }},0,\frac{\Lambda_{0}}{\mu_{0}},0,0\right). \end{array}$$

Following [29], we let

(9) $$\begin{array}{c} \tilde{g}\left(X^{*},Z\right)=\left({\tilde{g}}_{1}\left(X^{*},Z\right),{\tilde{g}}_{2}\left(X^{*},Z\right)\right), \end{array}$$

with

(10) $$\begin{array}{c} \left\{\begin{array}{c} {\tilde{g}}_{1}\left(X^{*},Z\right)=\frac{\beta_{C}\Lambda_{C}B_{C}}{\mu_{C}\left(\mu_{C}+\delta_{C}+\gamma_{C}\right)\left(B_{0}+B_{C}\right)},\\ {\tilde{g}}_{2}\left(X^{*},Z\right)=\frac{\beta_{\phi }\Lambda_{\phi }B_{c}}{\mu_{\phi }\left(\mu_{\phi }+k_{m}\right)}. \end{array}\right. \end{array}$$

We deduce that

(11) $$\begin{array}{c} h\left(X,Y,Z\right)=\left(h_{1}\left(X,Y,Z\right),h_{2}\left(X,Y,Z\right)\right), \end{array}$$

with

(12) $$\begin{array}{c} \left\{\begin{array}{c} h_{1}\left(X,Y,Z\right)=\frac{K_{0}B_{C}B_{m}}{\left(B_{0}+B_{c}\right)}+\alpha_{c}B_{c}-\alpha_{C}B_{C},\\ h_{2}\left(X,Y,Z\right)=\frac{K_{1}B_{C}}{\left(K_{3}+K_{2}B_{C}\right)}+K_{4}B_{c}-\left(\mu_{c}+\alpha_{c}\right)B_{c}, \end{array}\right. \end{array}$$

where

(13) $$\begin{array}{c} \left\{\begin{array}{c} K_{0}=\frac{\beta_{C}\Lambda_{C}\alpha_{c}}{\mu_{C}\left(\mu_{C}+\delta_{C}+\gamma_{C}\right)},\\ K_{1}=\frac{\beta_{C}\left(\Lambda_{C}-\mu_{C}\right)\left(\mu_{C}+\delta_{C}+\gamma_{C}\right)}{\Phi_{C}},\\ K_{2}=\beta_{C}\Lambda_{C}+\mu_{C}\left(\mu_{C}+\delta_{C}+\gamma_{C}\right),\\ K_{3}=\mu_{C}\left(\mu_{C}+\delta_{C}+\gamma_{C}\right)B_{0},\\ K_{4}=\frac{\beta_{\phi }\Lambda_{\phi }N_{m}k_{m}}{\mu_{\phi }\left(\mu_{\phi }+k_{m}\right)}. \end{array}\right. \end{array}$$

The matrix

(14) $$\begin{array}{c} A=D_{Z}h\left(X^{*},\tilde{g}\left(X^{*},0\right),0\right)=\left[\begin{array}{cc} -\alpha_{C} & \alpha_{c}\\ \frac{K_{1}}{K_{3}} & K_{4}-\left(\mu_{c}+\alpha_{c}\right) \end{array}\right], \end{array}$$

can be written in the form *A* = *M* − *D*, so that

(15) $$\begin{array}{c} M=\left[\begin{array}{cc} 0 & \alpha_{c}\\ \frac{K_{1}}{K_{3}} & K_{4} \end{array}\right],\\ D=\left[\begin{array}{cc} \alpha_{C} & 0\\ 0 & \left(\mu_{c}+\alpha_{c}\right) \end{array}\right]. \end{array}$$

The basic reproductive number is the spectral radius (dominant eigenvalue) of the matrix *T* = *MD*^−1^, that is,

(16) $$\begin{array}{c} R_{0}=\rho \left(T\right). \end{array}$$

Hence, in this case, the basic reproduction number of the embedded multiscale model (1) is expressed by the following quantity

(17) $$\begin{array}{c} R_{0}=\frac{1}{2}\left[R_{0c}+\sqrt{R_{0_{\text{C}}}^{2}+4R_{0C}}\right], \end{array}$$

with

(18) $$\begin{array}{c} R_{0c}=\frac{\beta_{\phi }\Lambda_{\phi }N_{m}k_{m}}{\mu_{\phi }\left(\mu_{\phi }+k_{m}\right)\left(\mu_{c}+\alpha_{c}\right)}, \end{array}$$

being a partial within-host basic reproduction number, and

(19) $$\begin{array}{c} R_{0C}=\frac{\beta_{C}\left(\Lambda_{C}-\mu_{C}\right)\alpha_{c}}{\alpha_{C}\mu_{C}\Phi_{C}\left(\mu_{c}+\alpha_{c}\right)}, \end{array}$$

being a partial between-host reproduction number.

Overall, we can conclude from expression (17) of the reproductive number that it is a function of both the within-host scale parameters and the between-host scale parameters. Therefore, the obtained results here show that the within-host scale and the between-host scale influence each other in a reciprocal way. We further make a use of the basic reproductive number (17) to test both the local and global stability of the disease-free equilibrium (*E*_0_) of the multiscale model system (1). We then established that if the basic reproductive number is less than a unity, then *E*_0_ is locally and globally asymptotically stable. Details of the local and global stability of *E*_0_ are given in the following next two subsections.

### 3.2. Stability of the Disease-Free Equilibrium

#### 3.2.1. Local Stability of the Disease-Free Equilibrium

In this subsection, we determine the local stability of DFE of the PTB multiscale model system (1). We linearize equations of the PTB multiscale model system (1) in order to obtain a Jacobian matrix. Then, we evaluate the Jacobian matrix of the system at the disease-free equilibrium (DFE),

(20) $$\begin{array}{c} E_{0}=\left(\frac{\Lambda_{C}}{\mu_{C}},0,0,0,\frac{\Lambda_{\phi }}{\mu_{\phi }},0,\frac{\Lambda_{0}}{\mu_{0}},0,0\right). \end{array}$$

The Jacobian matrix of the PTB multiscale model system (1) evaluated at the disease-free equilibrium state (DFE) is given by

(21) $$\begin{array}{c} J\left(E_{0}\right)=\left(\begin{array}{ccccccccc} -\mu_{C} & \gamma_{C} & -\frac{\beta_{C}\Lambda_{C}}{\mu_{C}B_{0}} & 0 & 0 & 0 & 0 & 0 & 0\\ 0 & -a_{0} & \frac{\beta_{C}\Lambda_{C}}{\mu_{C}B_{0}} & 0 & 0 & 0 & 0 & 0 & 0\\ 0 & 0 & -\alpha_{C} & \alpha_{c} & 0 & 0 & 0 & 0 & 0\\ 0 & 0 & A_{1} & -a_{1} & 0 & N_{m}k_{m} & 0 & 0 & 0\\ 0 & 0 & 0 & -\frac{\beta_{\phi }\Lambda_{\phi }}{\mu_{\phi }} & -\mu_{\phi } & 0 & 0 & 0 & 0\\ 0 & 0 & 0 & \frac{\beta_{\Phi }\Lambda_{\phi }}{\mu_{\phi }} & 0 & -a_{2} & 0 & 0 & 0\\ 0 & 0 & 0 & -\frac{\delta_{b}\Lambda_{0}}{\mu_{0}} & 0 & -\frac{\delta_{m}\Lambda_{0}}{\mu_{0}} & -\mu_{0} & 0 & 0\\ 0 & 0 & 0 & 0 & 0 & \frac{\theta_{1}\delta_{m}\Lambda_{0}}{\mu_{0}} & 0 & -\mu_{1} & 0\\ 0 & 0 & 0 & \frac{\theta_{2}\delta_{b}\Lambda_{0}}{\mu_{0}} & 0 & 0 & 0 & 0 & -\mu_{2}, \end{array}\right), \end{array}$$

where

(22) $$\begin{array}{c} \left\{\begin{array}{c} a_{0}=\left(\mu_{C}+\delta_{C}+\gamma_{C}\right),a_{1}=\left(\mu_{c}+\alpha_{c}\right),\\ a_{2}=\left(\mu_{\phi }+k_{m}\right),A_{1}=\frac{\beta_{C}\left(\Lambda_{C}-\mu_{C}\right)}{\Phi_{C}\mu_{C}B_{0}}. \end{array}\right. \end{array}$$

We consider stability of DFE by calculating the eigenvalues (*λ*_*s*_) of the Jacobian matrix given by equation (21). The characteristic equation for the eigenvalues is given by

(23) $$\begin{array}{c} Q_{0}\left[\lambda^{3}+\Phi_{1}\lambda^{2}+\Phi_{2}\lambda +\Phi_{3}\right]=0, \end{array}$$

where the coefficient *Q*_0_ is as follows:

(24) $$\begin{array}{c} Q_{0}=\left(-\mu_{C}-\lambda \right)\left(-\mu_{\phi }-\lambda \right)\left(-\mu_{0}-\lambda \right)\left(-\mu_{1}-\lambda \right)\left(-\mu_{2}-\lambda \right)\left(-a_{0}-\lambda \right). \end{array}$$

It can be easily noted from equation (23) that there are six negative eigenvalues (-*μ*_*C*_, -*μ*_*ϕ*_, -*μ*_0_, -*a*_0_, -*μ*_1_, and -*μ*_2_). Now in order to make conclusions about the stability of the DFE, we use the Routh-Hurwitz criteria to determine the sign of the remaining eigenvalues of the polynomial

(25) $$\begin{array}{c} \lambda^{3}+\Phi_{1}\lambda^{2}+\Phi_{2}\lambda +\Phi_{3}=0, \end{array}$$

where

(26) $$\begin{array}{c} \left\{\begin{array}{c} \Phi_{1}=\alpha_{C}+a_{1}+a_{2},\\ \Phi_{2}=\left(\alpha_{C}+a_{2}\right)a_{1}+\alpha_{C}a_{2}\left(1-R_{0C}\right),\\ \Phi_{3}=a_{1}a_{2}\left[R_{0c}+\alpha_{C}\left(1-R_{0C}\right)\right]. \end{array}\right. \end{array}$$

Using the Routh-Hurwitz stability criterion, the equilibrium state associated with the PTB multiscale model system (1) is stable if and only if the determinants of all the Hurwitz matrices associated with the characteristic equation (25) are positive, that is

(27) $$\begin{array}{c} \text{Det}\left(H_{j}\right)>0;j=1,2,3, \end{array}$$

where

(28) $$\begin{array}{c} \left\{\begin{array}{c} H_{1}=\left(\Phi_{1}\right);H_{2}=\left(\begin{array}{cc} \Phi_{1} & 1\\ \Phi_{3} & \Phi_{2} \end{array}\right),\\ H_{3}=\left(\begin{array}{ccc} \Phi_{1} & 1 & 0\\ \Phi_{3} & \Phi_{2} & \Phi_{1}\\ 0 & 0 & \Phi_{3} \end{array}\right). \end{array}\right. \end{array}$$

The Routh-Huiwitz criterion applied to expressions in equation (28) requires that the following conditions *C*1 and *C*2 be satisfied, in order to guarantee the local stability of the disease-free equilibrium point of the model system (1).

(29) $$\begin{array}{c} \left\{\begin{array}{cc} C1.\Phi_{1},\Phi_{2},\Phi_{3} & >0,\\ C2.\Phi_{1}\Phi_{2}-\Phi_{3} & >0. \end{array}\right. \end{array}$$

From equations (25) and (28), we note that all the coefficients *Φ*_1_, *Φ*_2_, and *Φ*_3_ of the polynomial *P*(*λ*) are greater than zero whenever *R*_0*C*_, *R*_0*c*_ < 1. And we also noted that the conditions above are satisfied if and only if *R*_0_ < 1. Hence, all the roots of the polynomial *P*(*λ*) are either negative or have negative real parts. The results are summarized in the following theorem.

**Theorem 1 .**

The disease-free equilibrium point of the model system (1) is locally asymptotically stable whenever *R*_0_ < 1.

#### 3.2.2. Global Stability of the Disease-Free Equilibrium

We determine the global stability of DFE of the PTB embedded multiscale model system (1) by using a next generation operator [29]. Thus, the system (1) can be rewritten in the form

(30) $$\begin{array}{c} \left\{\begin{array}{c} \frac{dX}{dt}=F\left(X,Z\right),\\ \frac{dY}{dt}=G\left(X,Z\right), \end{array}\right. \end{array}$$

where

- *X* = *S*_*C*_, *M*_*ϕ*_, *T*_0_, *T*_1_, *T*_2_ comprises of the uninfected components
- *Z* = *I*_*C*_, *B*_*C*_, *B*_*c*_, *I*_*m*_ comprises of infected and infectious components

We let

(31) $$\begin{array}{c} E_{0}=\left(X^{*},0\right)=\left(\frac{\Lambda_{C}}{\mu_{C}},0,0,0,\frac{\Lambda_{\phi }}{\mu_{\phi }},0,\frac{\Lambda_{0}}{\mu_{0}},0,0\right), \end{array}$$

denote the disease-free equilibrium (DFE) of the embedded multiscale model system (1). For *E*_0_ to be globally asymptotically stable, the following conditions (H1) and (H2) must be satisfied.

(H1.) *dX*/*dt* = *F*(*X*, 0) is globally asymptotically stable (g.a.s)
(H2.) $G\left(X,Z\right)=AZ-\hat{G}\left(X,Z\right)$, $\hat{G}\left(\left(X,Z\right)\right.\geq 0$ for (*X*, *Z*) ∈ *R*_+_^9^ where *A* = *D*_*Z*_*G*(*X*^∗^, 0) is an M-matrix and *R*_+_^9^ is the region where the model makes biological sense

In this case

(32) $$\begin{array}{c} F\left(X,0\right)=\left[\begin{array}{c} \Lambda_{C}-\mu_{C}S_{C}\\ \Lambda_{\phi }-\mu_{\phi }M_{\phi }\\ 0\\ 0 \end{array}\right], \end{array}$$

and the matrix *A* is given by

(33) $$\begin{array}{c} A=\left[\begin{array}{cccc} -\left(\mu_{C}+\delta_{C}+\gamma_{C}\right) & \frac{\beta_{C}\Lambda_{C}}{B_{0}\mu_{C}} & 0 & 0\\ 0 & -\alpha_{C} & \alpha_{c} & 0\\ 0 & \frac{\beta_{\text{C}}\left(\Lambda_{C}-\mu_{C}\right)}{B_{0}\Phi_{C}\mu_{C}} & -\left(\alpha_{c}+\mu_{c}\right) & N_{m}k_{m}\\ 0 & 0 & \frac{\beta_{\phi }\Lambda_{\phi }}{\mu_{\phi }} & -\left(\mu_{\phi }+k_{m}\right) \end{array}\right], \end{array}$$

with $\hat{G}\left(X,Z\right)$ given by

(34) $$\begin{array}{c} \hat{G}\left(X,Z\right)=\left[\begin{array}{c} \left(\frac{\Lambda_{C}}{B_{0}\mu_{C}}-\frac{S_{C}}{B_{0}+B_{C}}\right)\beta_{C}B_{C}\\ 0\\ 0\\ \left(\frac{\Lambda_{\phi }}{\mu_{\phi }}-M_{\phi }\right)\beta_{\phi }B_{c}+\gamma_{m}T_{1}I_{m}. \end{array}\right]. \end{array}$$

It is clear that $\hat{G}\left(X,Z\right)\geq 0$ for all (*X*, *Z*) ∈ *R*_+_^9^, since (*Λ*_*C*_/*μ*_*C*_*B*_0_) ≥ (*S*_*C*_/(*B*_0_ + *B*_*C*_)) and (*Λ*_*ϕ*_/*μ*_*ϕ*_) ≥ *M*_*ϕ*_. It is also clear that *A* is an M-matrix, since the off diagonal elements of *A* are nonnegative. We state a theorem which summarizes the above result.

**Theorem 2 .**

The disease-free equilibrium of model system (1) is globally asymptotically stable if *R*_0_ < 1, and the assumptions (H1) and (H2) are satisfied.

### 3.3. The Endemic Equilibrium and Its Stability

#### 3.3.1. The Existence of the Endemic Equilibrium State

The endemic equilibrium state of the multiscale model system (1) is obtained by setting the left-hand side of the model to zero. Letting

(35) $$\begin{array}{c} E^{*}=\left(S_{C}^{*},I_{C}^{*},B_{C}^{*},B_{c}^{*},M_{\phi }^{*},I_{m}^{*},T_{0}^{*}T_{1}^{*},T_{2}^{*}\right), \end{array}$$

be the endemic solution for the multiscale model system (1), we can then estimate the disease burden of PTB in ruminants when the disease has reached its endemic level. We achieve this by considering the dependences of endemic values of the PTB disease variables *S*_*C*_^∗^, *I*_*C*_^∗^, *B*_*C*_^∗^, *B*_*c*_^∗^, *M*_*ϕ*_^∗^, *I*_*m*_^∗^, *T*_0_^∗^, *T*_1_^∗^, *T*_2_^∗^. The endemic value of susceptible humans is given by

(36) $$\begin{array}{c} S_{C}^{*}=\frac{\Lambda_{C}+\gamma_{C}I_{C}^{*}}{\lambda_{C}^{*}+\mu_{C}}. \end{array}$$

From (36), we note that the susceptible ruminant population at endemic equilibrium is given by the average time of stay in the susceptible class and the rate at which new susceptible individuals are entering the susceptible class at a constant rate *Λ*_*C*_ as well as infected ruminant individuals entering the class through recovery at a rate *γ*_*C*_. Susceptible ruminants leave the susceptible class either through infection or death. The endemic value of infected ruminants is given by

(37) $$\begin{array}{c} I_{C}^{*}=\frac{\lambda_{C}^{*}S_{C}^{*}}{\mu_{C}+\delta_{C}+\gamma_{C}}. \end{array}$$

We note from (37) that the population of infected ruminants at the endemic equilibrium point is determined by the average time of stay in the infected class, the rate at which susceptible ruminants become infected and the density of susceptible ruminants. The endemic value of between-host scale MAP bacterial load in the environment at the equilibrium point is given by

(38) $$\begin{array}{c} B_{C}^{*}=\frac{\alpha_{c}B_{c}^{*}\left(I_{C}^{*}+1\right)}{\alpha_{C}}. \end{array}$$

From equation (38), we note that the between-host MAP bacterial load in the environment at the equilibrium point is equal to the average life-span of the bacteria in the environment and the rate of excretion of the average number of the within-host MAP bacterial load by each infected ruminant individual into the environment. We also note that this expression provides a link between the dynamics of the within-host MAP bacteria load and the transmission dynamics of the disease at the ruminant population level. The endemic value of within-host scale MAP bacterial load within a single infected ruminant is given by

(39) $$\begin{array}{c} B_{c}^{*}=\frac{\lambda_{c}^{*}S_{c}^{*}+N_{m}k_{m}I_{m}^{*}}{\left(\alpha_{c}+\mu_{c}\right)}. \end{array}$$

We note from (39) that the population of within-host MAP bacteria within a single infected ruminant at endemic equilibrium point is determined by the average dose of the between-host bacterial load in the environment are ingested and the average life-span of within-host bacterial load at the site of infection within an infected ruminant and the average number rate of the within-host MAP bacilli bacteria produced upon bursting of infected macrophage cells at a site of infection. We also note that this expression provides a link between the dynamics of the between-host MAP bacteria load in the environment and the within-host infection dynamics within a single infected ruminant. The value of susceptible macrophage population within a single infected ruminant at equilibrium point is given by

(40) $$\begin{array}{c} M_{\phi }^{*}=\frac{\Lambda_{\phi }}{\beta_{\phi }B_{c}^{*}+\mu_{\phi }}. \end{array}$$

From (40), we note that susceptible macrophage population at endemic equilibrium is proportional to the average time of stay in susceptible macrophage class and the rate at which new susceptible macrophage is supplied into the susceptible macrophage class at the site of infection within an infected ruminant. The endemic value of infected macrophage population is given by

(41) $$\begin{array}{c} I_{m}^{*}=\frac{\beta_{\phi }B_{c}^{*}M_{\phi }^{*}}{k_{m}+\mu_{\phi }+\gamma_{m}T_{1}^{*}}. \end{array}$$

We also note from (41) that infected macrophage population at the endemic equilibrium point is proportional to the average time of stay in the infected macrophage class at the site of infection, the rate at which susceptible macrophages become infected and the density of susceptible macrophages. The endemic value of naive CD4 T cell population within a single infected ruminant at the site of infection is given by

(42) $$\begin{array}{c} T_{0}^{*}=\frac{\Lambda_{0}}{\delta_{m}I_{m}^{*}+\delta_{b}B_{c}^{*}+\mu_{0}}. \end{array}$$

The average population of naive immune response cells at a site of infection within an infected human at endemic equilibrium point is equal to the average life-span of naive CD4 T cells and the supply rate of naive CD4 T cells into a site of infection from the source within an infected ruminant body. The endemic value of a single ruminant MAP-specific immune response Th1 effector cells within a single infected ruminant at the site of infection is given by

(43) $$\begin{array}{c} T_{1}^{*}=\frac{\theta_{1}\delta_{m}I_{m}^{*}T_{0}^{*}}{\mu_{1}}. \end{array}$$

The average population of MAP-specific immune response Th1 effector cells within an infected ruminant is proportional to the differential rate of naive CD4 T cells into the class of MAP-specific immune response cell Th1 effector population after a detection of infected macrophage cells at the site of infection. The endemic value of a single ruminant MAP-specific immune response Th2 effector cell within a single infected ruminant at the site of infection is given by

(44) $$\begin{array}{c} T_{2}^{*}=\frac{\theta_{2}\delta_{b}B_{c}^{*}T_{0}^{*}}{\mu_{2}}. \end{array}$$

We note from (44) that the MAP-specific immune response Th1 effector cell population within a single infected ruminant at equilibrium point is proportional to the differential rate of naive CD4 T cells into the class of MAP-specific immune response Th2 effector population after a detection of the within-host scale MAP bacterial load at the site of infection.

From the endemic equilibrium values of the model system (1) given by expressions (36)–(44), we can easily deduce that the between-host scale expression *B*_*C*_^∗^ depends on both the within-host scale and the between-host scale disease variables, while the within-host scale expression *B*_*c*_^∗^ is determined by both the within-host and the between-host disease variables. Therefore, the obtained results here show that the within-host scale and the between-host scale dynamics influence each other in a reciprocal way. The next section is the analysis for the stability of the endemic equilibrium (*E*^∗^) of the multiscale model system (1), where we use the center manifold theory [30].

#### 3.3.2. Local Stability of the Endemic Equilibrium State

In this subsection, we study the local asymptotic stability of the endemic steady state of the model system (1) by using the center manifold theory described in [30]. In this case, we employ center manifold theory by making the following change of variables: letting *S*_*C*_ = *x*_1_, *I*_*C*_ = *x*_2_, *B*_*C*_ = *x*_3_, *B*_*c*_ = *x*_4_, *M*_*ϕ*_ = *x*_5_, *I*_*m*_ = *x*_6_, *T*_0_ = *x*_7_, *T*_1_ = *x*_8_, and *T*_2_ = *x*_9_. We also use the vector notation *x* = (*x*_1_, *x*_2_, *x*_3_, *x*_4_, *x*_5_, *x*_6_, *x*_7_, *x*_8_, *x*_9_)^*T*^ so that the model system (1) can be written in the form

(45) $$\begin{array}{c} \frac{dx}{dt}=f\left(x,\beta^{*}\right), \end{array}$$

where

(46) $$\begin{array}{c} f=\left(f_{1},f_{2},f_{3},f_{4},f_{5},f_{6},f_{7},f_{8},f_{9}\right). \end{array}$$

Therefore, model system (1) can be rewritten as follows:

(47) $$\begin{array}{c} \left\{\begin{array}{cc} 1. & {\dot{x}}_{1}=\Lambda_{C}-\frac{\beta_{C}x_{3}\left(t\right)x_{1}\left(t\right)}{B_{0}+x_{3}\left(t\right)}-\mu_{C}x_{1}\left(t\right)+\gamma_{C}x_{2}\left(t\right),\\ 2. & {\dot{x}}_{2}=\frac{\beta_{C}x_{3}\left(t\right)x_{1}\left(t\right)}{B_{0}+x_{3}\left(t\right)}-\left[\mu_{C}+\delta_{C}+\gamma_{C}\right]x_{2}\left(t\right),\\ 3. & {\dot{x}}_{3}=\alpha_{c}x_{4}\left(t\right)\left(x_{2}\left(t\right)+1\right)-\alpha_{C}x_{3}\left(t\right),\\ 4. & {\dot{x}}_{4}=\frac{\beta_{C}x_{3}\left(t\right)\left(x_{1}\left(t\right)-1\right)}{\left(B_{0}+x_{3}\left(t\right)\right)\Phi_{C}\left(x_{2}+1\right)}+N_{m}k_{m}x_{6}\left(t\right)-\left[\mu_{c}+\alpha_{c}\right]x_{4}\left(t\right),\\ 5. & {\dot{x}}_{5}=\Lambda_{\phi }-\beta_{\phi }x_{5}\left(t\right)x_{4}\left(t\right)-\mu_{\phi }x_{5}\left(t\right),\\ 6. & {\dot{x}}_{6}=\beta_{\phi }x_{5}\left(t\right)x_{4}\left(t\right)-\gamma_{m}x_{8}\left(t\right)x_{6}\left(t\right)-\left[k_{m}+\mu_{\phi }\right]x_{6}\left(t\right),\\ 7. & {\dot{x}}_{7}=\Lambda_{0}-\left[\delta_{m}x_{6}\left(t\right)+\delta_{b}x_{4}\left(t\right)\right]x_{7}\left(t\right)-\mu_{0}x_{7}\left(t\right),\\ 8. & {\dot{x}}_{8}=\theta_{1}\delta_{m}x_{6}\left(t\right)x_{7}\left(t\right)-\mu_{1}x_{8}\left(t\right),\\ 9. & {\dot{x}}_{9}=\theta_{2}\delta_{b}x_{4}\left(t\right)x_{7}\left(t\right)-\mu_{2}x_{9}\left(t\right). \end{array}\right. \end{array}$$

The method involves evaluating the Jacobian matrix of the system (47) at the disease-free equilibrium *E*^0^ denoted by *J*(*E*^0^). The Jacobian matrix associated with the system of equation (47) evaluated at the disease-free equilibrium (*E*_0_) is given by

(48) $$\begin{array}{c} J\left(E_{0}\right)=\left(\begin{array}{ccccccccc} -\mu_{C} & \gamma_{C} & -\frac{\beta_{C}\Lambda_{C}}{\mu_{C}B_{0}} & 0 & 0 & 0 & 0 & 0 & 0\\ 0 & -z_{0} & \frac{\beta_{C}\Lambda_{C}}{\mu_{C}B_{0}} & 0 & 0 & 0 & 0 & 0 & 0\\ 0 & 0 & -\alpha_{C} & \alpha_{c} & 0 & 0 & 0 & 0 & 0\\ 0 & 0 & q_{1} & -z_{1} & 0 & N_{m}k_{m} & 0 & 0 & 0\\ 0 & 0 & 0 & -\frac{\beta_{\phi }\Lambda_{\phi }}{\mu_{\phi }} & -\mu_{\phi } & 0 & 0 & 0 & 0\\ 0 & 0 & 0 & \frac{\beta_{\phi }\Lambda_{\phi }}{\mu_{\phi }} & 0 & -z_{2} & 0 & 0 & 0\\ 0 & 0 & 0 & -\frac{\delta_{b}\Lambda_{0}}{\mu_{0}} & 0 & -\frac{\delta_{m}\Lambda_{0}}{\mu_{0}} & -\mu_{0} & 0 & 0\\ 0 & 0 & 0 & 0 & 0 & \frac{\theta_{1}\delta_{m}\Lambda_{0}}{\mu_{0}} & 0 & -\mu_{1} & 0\\ 0 & 0 & 0 & \frac{\theta_{2}\delta_{b}\Lambda_{0}}{\mu_{0}} & 0 & 0 & 0 & 0 & -\mu_{2}, \end{array}\right), \end{array}$$

where

(49) $$\begin{array}{c} \left\{\begin{array}{c} z_{0}=\left(\mu_{C}+\delta_{C}+\gamma_{C}\right),z_{1}=\left(\mu_{c}+\alpha_{c}\right),\\ z_{2}=\left(\mu_{\phi }+k_{m}\right),q_{1}=\frac{\beta_{C}\left(\Lambda_{C}-\mu_{C}\right)}{\Phi_{C}\mu_{C}B_{0}}. \end{array}\right. \end{array}$$

By using the similar approach as in [29], therefore the basic reproductive number of model system (47) is

(50) $$\begin{array}{c} R_{0}=\frac{1}{2}\left[R_{0c}+\sqrt{R_{0c}^{2}+4R_{0C}}\right], \end{array}$$

where

(51) $$\begin{array}{c} R_{0c}=\frac{\beta_{\phi }\Lambda_{\phi }N_{k}k_{m}}{\mu_{\phi }\left(\mu_{\phi }+k_{m}\right)\left(\mu_{c}+\alpha_{c}\right)},\\ R_{0C}=\frac{\beta_{C}\left(\Lambda_{C}-\mu_{C}\right)\alpha_{c}}{\alpha_{C}B_{0}\mu_{C}\left(\mu_{c}+\alpha_{c}\right)\Phi_{C}}. \end{array}$$

Now let us consider *β*_*ϕ*_ = *kβ*_*C*_, regardless of whether *k* ∈ (0, 1) or *k* ≥ 1 and let *β*_*C*_ = *β*^∗^ be a bifurcation parameter of the model system (47). Considering *R*_0_ = 1 and solve for *β*^∗^ in equation (50), we obtain

(52) $$\begin{array}{c} \beta^{*}=\frac{\left(\mu_{c}+\alpha_{c}\right)\mu_{\phi }\left(\mu_{\phi }+k_{m}\right)\alpha_{C}B_{0}\mu_{C}\Phi_{C}}{k\Lambda_{\phi }N_{m}k_{m}\alpha_{C}\mu_{C}B_{0}\mu_{C}\Phi_{C}+\alpha_{c}\left(\Lambda_{C}-\mu_{C}\right)\mu_{\phi }\left(\mu_{\phi }+k_{m}\right)}. \end{array}$$

We can easily note that the linearized system of the transformed equation (47) with bifurcation point *β*^∗^ has a simple zero eigenvalue. Hence, the center manifold theory [30] can be used to analyze the dynamics of (2.48) near *β*_*C*_ = *β*^∗^. We, therefore, apply Theorem 4.1 in Castillo-Chavez and Song [31] as stated in Appendix B for convenience. For us to apply Theorem B.1 in Appendix B, the following computations are necessary (it should be noted that we are using *β*^∗^ as the bifurcation parameter, in place of *ϕ* in Theorem B.1).

*Eigenvectors ofJ*_*β* ^∗^_: For the case when *R*_0_ = 1, it can be shown that the Jacobian matrix of (48) at *β*_*C*_ = *β*^∗^ (denoted by *J*_*β*^∗^_) has a right eigenvector associated with the zero eigenvalue given by

(53) $$\begin{array}{c} u={\left[u_{1},u_{2},u_{3},u_{4},u_{5},u_{6},u_{7},u_{8},u_{9}\right]}^{T}, \end{array}$$

where

(54) $$\begin{array}{c} \left\{\begin{array}{c} u_{1}=-\frac{\beta^{*}\Lambda_{C}\left(1-\gamma_{C}\right)}{\mu_{C}^{2}B_{0}\alpha_{C}},u_{2}=\frac{\alpha_{c}\beta^{*}\Lambda_{C}}{B_{0}\mu_{C}\left(\mu_{C}+\delta_{C}+\gamma_{C}\right)\alpha_{C}},u_{3}=\frac{\alpha_{c}}{\alpha_{C}},\\ u_{4}=1,u_{5}=-\frac{k\beta^{*}\Lambda_{\phi }}{\mu_{\phi }^{2}},u_{6}=\frac{k\beta^{*}\Lambda_{\Phi }}{\mu_{\phi }\left(\mu_{\phi }+k_{m}\right)},\\ u_{7}=-\left[\frac{\delta_{b}\Lambda_{0}}{\mu_{0}^{2}}+\frac{\delta_{m}\Lambda_{0}k\beta^{*}\Lambda_{\Phi }}{\mu_{0}^{2}\left(\mu_{\phi }+k_{m}\right)\mu_{\phi }}\right],u_{8}=\frac{\theta_{1}\delta_{m}\Lambda_{0}k\beta^{*}\Lambda_{\phi }}{\mu_{0}\left(\mu_{\phi }+k_{m}\right)\mu_{\phi }\mu_{1}},u_{9}=\frac{\theta_{2}\delta_{b}\Lambda_{0}}{\mu_{0}\mu_{2}}. \end{array}\right. \end{array}$$

In addition, the left eigenvector of the Jacobian matrix in (48) associated with the zero eigenvalue at *β*_*C*_ = *β*^∗^ is given by

(55) $$\begin{array}{c} v={\left[v_{1},v_{2},v_{3},v_{4},v_{5},v_{6},v_{7},v_{8},v_{9}\right]}^{T}, \end{array}$$

where

(56) $$\begin{array}{c} \left\{\begin{array}{c} v_{1}=0,v_{2}=0,v_{3}=\frac{\beta^{*}\left(\Lambda_{C}-\mu_{C}\right)}{\alpha_{C}\mu_{C}\Phi_{C}B_{0}},\\ v_{4}=1,v_{5}=0,v_{6}=\frac{N_{m}k_{m}}{\left(\mu_{\phi }+k_{m}\right)},\\ v_{7}=0,v_{8}=0,v_{9}=0. \end{array}\right. \end{array}$$

Computation of bifurcation parameters *a* and *b*:

We evaluate the nonzero second order mixed derivatives of **f** with respect to the variables and *β*^∗^ in order to determine the signs of *a* and *b*. The sign of *a* is associated with the following nonvanishing partial derivatives of **f**:

(57) $$\begin{array}{c} \left\{\begin{array}{c} \frac{\partial^{2}f_{1}}{\partial x_{3}^{2}}=\frac{2\beta^{*}\Lambda_{C}}{B_{0}^{2}\mu_{C}},\\ \frac{\partial^{2}f_{2}}{\partial x_{3}^{2}}=-\frac{2\beta^{*}\Lambda_{C}}{B_{0}^{2}\mu_{C}},\\ \frac{\partial^{2}f_{3}}{\partial x_{3}^{2}}=-\frac{2\beta^{*}\left(\Lambda_{C}-\mu_{C}\right)}{B_{0}^{2}\mu_{C}\Phi_{C}}. \end{array}\right. \end{array}$$

The sign of *b* is associated with the following nonvanishing partial derivatives of **f**:

(58) $$\begin{array}{c} \left\{\begin{array}{c} \frac{\partial^{2}f_{1}}{\partial x_{3}\partial \beta^{*}}=-\frac{\Lambda_{C}}{\mu_{C}B_{0}},\\ \frac{\partial^{2}f_{2}}{\partial x_{3}\partial \beta^{*}}=\frac{\Lambda_{C}}{\mu_{C}B_{0}},\\ \frac{\partial^{2}f_{4}}{\partial x_{3}\partial \beta^{*}}=\frac{\left(\Lambda_{C}-\mu_{C}\right)}{\mu_{C}B_{0}\Phi_{C}},\\ \frac{\partial^{2}f_{5}}{\partial x_{4}\partial \beta^{*}}=-\frac{\Lambda_{\phi }}{\mu_{\phi }},\\ \frac{\partial^{2}f_{6}}{\partial x_{4}\partial \beta^{*}}=\frac{k\Lambda_{\phi }}{\mu_{\phi }}. \end{array}\right. \end{array}$$

Substituting expressions (54) and (56), (57) into equation (B.2), we get

(59) $$\begin{array}{c} \left\{a=u_{1}v_{3}^{2}\frac{\partial^{2}f_{1}}{\partial x_{3}^{2}}+u_{2}v_{3}^{2}\frac{\partial^{2}f_{2}}{\partial x_{3}^{2}}+u_{4}v_{3}^{2}\frac{\partial^{2}f_{4}}{\partial x_{3}^{2}},=u_{1}v_{3}^{2}\left[\frac{2\beta^{*}\Lambda_{C}}{B_{0}^{2}\mu_{C}}\right]+u_{2}v_{3}^{2}\left[\frac{-2\beta^{*}\Lambda_{C}}{B_{0}^{2}\mu_{C}}\right]+u_{4}v_{3}^{2}\left[\frac{-2\beta^{*}\left(\Lambda_{C}-\mu_{C}\right)}{\Phi_{C}B_{0}^{2}\mu_{C}}\right],=\frac{2\beta^{*}\Lambda_{C}}{B_{0}^{2}\mu_{C}}.v_{3}^{2}\left[u_{1}-u_{2}\right]-u_{4}v_{3}^{2}\left[\frac{2\beta^{*}\left(\Lambda_{C}-\mu_{C}\right)}{\Phi_{C}B_{0}^{2}\mu_{C}}\right]<0,\right. \end{array}$$

since (*u*_1_ − *u*_2_) < 0, *u*_4_ > 0, and *v*_3_ > 0.

Similarly, substituting expressions (54) and (56) and (58) into equation (B.2), we get

(60) $$\begin{array}{c} \left\{b=u_{1}v_{3}\frac{\partial^{2}f_{1}}{\partial x_{3}\partial \beta^{*}}+u_{2}v_{3}\frac{\partial^{2}f_{2}}{\partial x_{3}\partial \beta^{*}}+u_{4}v_{3}\frac{\partial^{2}f_{4}}{\partial x_{3}\partial \beta^{*}}+u_{5}v_{4}\frac{\partial^{2}f_{4}}{\partial x_{10}\partial \beta^{*}}+u_{6}v_{4}\frac{\partial^{2}f_{6}}{\partial x_{4}\partial \beta^{*}},=v_{3}\left[\frac{\Lambda_{C}}{B_{0}\mu_{C}}.u_{2}-\frac{\Lambda_{C}}{B_{0}\mu_{C}}.u_{1}+\frac{\left(\Lambda_{C}-\mu_{C}\right)}{\Phi_{C}B_{0}\mu_{C}}.u_{4}\right]+v_{4}\left[\frac{k\Lambda_{\phi }}{\mu_{\phi }}.u_{6}-\frac{k\Lambda_{\phi }}{\mu_{\phi }}.u_{5}\right],=\frac{\Lambda_{C}}{B_{0}\mu_{C}}.v_{3}\left[u_{2}-u_{1}\right]+\frac{\left(\Lambda_{C}-\mu_{C}\right)}{\Phi_{C}B_{0}\mu_{C}}.v_{3}u_{4}+\frac{k\Lambda_{\phi }}{\mu_{\phi }}.v_{4}\left[u_{6}-u_{5}\right]>0,\right. \end{array}$$

since (*u*_2_ − *u*_1_) > 0, (*u*_6_ − *u*_5_) > 0, *u*_4_ > 0, and *v*_3_ > 0.

Thus, *a* < 0 and *b* > 0. Using Theorem B.1, item (iv), we have established the following result which only holds for *R*_0_ > 1 but close to 1.

**Theorem 3 .**

The endemic equilibrium guaranteed by Theorem B.1 is locally asymptotically stable for *R*_0_ > 1 near 1.

## 4. Numerical Simulations and Sensitivity Analysis of the PTB Multiscale Model

In this section, we present some numerical simulations that demonstrate the reciprocal influence between the MAP replication process at the within-host scale and the MAP transmission process of PTB infection using numerical simulations of the embedded multiscale model. Numerical simulations of the model system (1) are carried out using a Python program version V 2.6 in windows operation system (Windows 10). The program uses a package odeint function in the python-scipy that integrate or solve any system of differential equations. We also perform some sensitivity analysis of the model basic reproductive number on the variation of the model parameters. The numerical values of the parameters used in the numerical simulations and sensitivity analysis are given in Table 2. In the next two subsections are the numerical simulation results obtained from the PTB multiscale model system (1).

### 4.1. The Influence of Between-Host Scale on the Within-Host PTB Disease Dynamics

In this subsection, we illustrate using numerical simulations the effect of the between-host scale submodel parameters on the within-host scale submodel variables of the embedded multiscale model (1). Figures 2–4 show the impact of variation of four between-host scale parameters (*β*_*C*_, *α*_*C*_, *B*_0_) on the dynamics of four selected key with-host scale variables (*I*_*m*_, *B*_*c*_, *T*_1_, *T*_2_).

Figure 2 shows graphs of numerical solutions of the model system (1) showing propagation of (a) infected macrophage population, (b) within-host scale MAP bacteria population, (c) MAP-specific Th1 immune response cells, and (d) MAP-specific Th2 immune response cells for different values of between-host scale transmission rate *β*_*C*_: *β*_*C*_ =0.00027, *β*_*C*_ =0.0027, and *β*_*C*_ =0.027. The results show that the variation in the infection rate at the between-host scale influence the dynamics of the disease at the within-host scale only within a period of about 50 days. But after that, the dynamics of the disease reach an endemic level. Therefore, this implies that different initial inoculum values converge to the same endemic state after a period of about 50 days. This confirms that for a pathogen with a replication cycle the superinfection only influences the within-host scale PTB population dynamics at the start of the infection.

Figure 3 illustrates the solution profile of the population of (a) infected macrophages, (b) within-host scale MAP bacteria, (c) MAP-specific Th1 immune response cells, and (d) MAP-specific Th2 immune response cells for different values of natural death rate of MAP bacilli in the environment *α*_*C*_: *α*_*C*_ =0.18, *α*_*C*_ =0.018, and *α*_*C*_ =0.0018. The results in Figure 3 show that the variation in the MAP bacilli death rate at the between-host scale influences the dynamics of the disease at the within-host scale only within a period of about 50 days. But after that, the dynamics of the disease reach an endemic level. Therefore, this also implies that different MAP bacilli death rate values converge to the same endemic state after a period of about 50 days. This also confirms that the superinfection only influences the within-host PTB population dynamics at the start of the infection and further confirms that as the between-host scale MAP bacilli decay rate increases, the time to reach the endemic state also increases.

Figure 4 shows the solution profile of the (a) infected macrophage population, (b) within-host scale MAP bacteria population, (c) MAP-specific Th1 immune response cells, and (d) MAP-specific Th2 immune response cells for different values of bacteria half saturation constant *B*_0_: *B*_0_ = 1000, *B*_0_ = 10000, and *B*_0_ = 100000. In Figure 4, the results show that the variation in the saturation rate of bacteria at the between-host scale influences the dynamics of the disease at the within-host scale only within a period of about 50 days. But after that, the dynamics of the disease reaches an endemic level. Therefore, this again implies that different saturation rates of bacteria values converge to the same endemic state after a period of about 50 days. This also confirms that for a pathogen with a replication cycle superinfection only influences the within-host scale PTB population dynamics at the start of the infection. This again confirms that as the initial inoculum increases, the time to reach the endemic state in the population of the within-host scale MAP bacteria also increases.

### 4.2. The Influence of Within-Host Scale on the Between-Host PTB Disease Dynamics

This subsubsection highlights some numerical assessment results of the influence of the within-host submodel parameters on the between-host submodel PTB transmission dynamics. Figures 5–7 show the impact in the variation of three within-host parameters (*α*_*c*_, *N*_*m*_, *μ*_*c*_) on the dynamics of three key between-host variables (*S*_*C*_, *I*_*C*_, *B*_*C*_).

Figure 5 shows graphs of numerical solutions of the model system (1) showing propagation of (a) population of susceptible ruminant (*S*_*C*_), (b) population of infected ruminant (*I*_*C*_), and (c) between-host MAP bacterial load (*B*_*C*_) for different values of excretion rate of within-host MAP bacilli into the environment *α*_*c*_: *α*_*c*_ = 0.001, *α*_*c*_ = 0.01, and *α*_*c*_ = 0.1. The results show that an increase of excretion rate of the within-host bacterial load into the physical environment by each infected ruminant individual has important public health effect at the ruminant population-level in that there is a noticeable increase in the between-host MAP bacteria *B*_*C*_ and population of infected ruminant *I*_*C*_ as well as decrease in the population of susceptible ruminant *S*_*C*_. This confirms that within-host parameters continuously influence the between-host PTB population dynamics throughout the infection.

Figure 6 shows graphs of numerical solutions of the model system (1) showing variation of (a) population of susceptible ruminants (*S*_*C*_), (b) population of infected ruminants (*I*_*C*_), and (c) between-host MAP bacterial load (*B*_*C*_) for different values of within-host scale MAP bacteria produced per bursting infected macrophage cell *N*_*m*_: *N*_*m*_ = 10, *N*_*m*_ = 100, and *N*_*m*_ = 1000. This shows that as the average replication rate of the within-host scale MAP bacilli bacteria for an infected macrophage cell at individual ruminant level increases, transmission of PTB infection at herd-level of ruminants also increases. This again confirms that within-host scale parameters continuously influence the between-host scale PTB population dynamics throughout the infection.

Figure 7 illustrates the solution profile of the multiscale model (1) showing variations of (a) population of susceptible ruminants (*S*_*C*_), (b) population of infected ruminants (*I*_*C*_), and (c) between-host scale MAP bacterial load (*B*_*C*_) for different values of natural death rate of within-host scale MAP bacilli at the site of infection within an infected ruminant *μ*_*c*_: *μ*_*c*_ = 0.3, *μ*_*c*_ = 0.025, and *μ*_*c*_ = 0.003. The results in Figure 7 show that as the death rate of the within-host scale MAP bacilli increases, there is a noticeable decrease in the between-host scale MAP bacterial load *B*_*C*_ and population of infected ruminants *I*_*C*_ as well as increase in population of susceptible ruminants *S*_*C*_. This further confirms that within-host scale parameters continuously influence the between-host scale PTB population dynamics throughout the infection.

Overall, the results in Figures 2–7 show that during the dynamics for PTB infection in ruminants, once the infection has successfully established at the within-host scale, the contribution of superinfection to the total pathogen load at this scale domain becomes negligible compared to the contribution of the pathogen replication. However, at the between-host scale, the dynamics of populations (*S*_*C*_, *I*_*C*_, *B*_*C*_) implicated in the spread of PTB are significantly sensitive to the variation of the three selected within-host scale parameters (*α*_*c*_, *μ*_*c*_, and *N*_*m*_), particularly the decay rate *μ*_*c*_ of the within-host scale MAP bacteria. We also performed sensitivity analysis of the PTB disease transmission metric to the parameters of the multiscale model system (1). In what follow, we present the sensitivity analysis results of the PTB disease transmission metric (i.e., the basic reproductive number) to the variation of the multiscale model system (1)'s parameters.

### 4.3. Sensitivity Analysis

In this section, we carry out sensitivity analysis on the basic reproductive number to evaluate the relative change in PTB disease dynamics metric when the within-host scale and between-host scale parameters of the multiscale model system (1) change. We achieve this by using Latin hypercube sampling (LHS) and partial rank correlation coefficients (PRCCs). The PTB disease dynamics metric used to characterize disease dynamics in this study is the basic reproductive number (*R*_0_) obtained from the multiscale model (1). We used 1000 simulations per run to investigate the impact of each of the multiscale model system (1)'s parameters. The results of the assessment of the sensitivity of the PTB basic reproductive number (*R*_0_) to the baseline PTB multiscale model system (1) parameters are shown in the Tornado plot, Figure 8. From Figure 8, we notice that some of the model parameters have positive PRCCs while some have negative PRCCs. Thus, parameters with positive PRCCs will increase *R*_0_ when they are increased, whereas parameters with negative PRCCs will decrease *R*_0_ when they are increased. For instance, increasing parameter like *N*_*m*_ increases the value of *R*_0_, and also increasing parameters like *μ*_*c*_ reduces the value of *R*_0_.

Therefore, from Figure 8, we make the following deductions:

- The most sensitive parameters to the PTB disease dynamics metric (*R*_0_) are *N*_*m*_, *k*_*m*_, *μ*_*ϕ*_, *μ*_*c*_, and *β*_*ϕ*_, with all being the within-host scale PTB disease dynamics. This implies that care should be taken in improving the accuracy of these five within-host scale parameters during data collection if the validity and utility of the multiscale model of PTB disease dynamics given by (1) is to be improved. From the assessment of the sensitivity of *R*_0_ to two additional parameters that we might have the most control over (*N*_*m*_ and *μ*_*c*_), we note that *R*_0_ is also significantly sensitive to all these two within-host scale parameters while having the highest sensitivity to *N*_*m*_. We conclude that administration of PTB drug treatment that kill and restrict bacteria cell replication at within-host scale will likely yield the highest benefits in reducing the transmission of PTB at between-host scale
- The least sensitive parameters to the PTB health intervention metric (R0) are *β*_*C*_, *Λ*_*C*_, *α*_*C*_, *μ*_*C*_, *Λ*_*ϕ*_, *B*_0_, *Φ*_*C*_, and *α*_*c*_. This indicates that the multiscale model system for PTB transmission dynamics given by (1) is robust to these parameters. We note from the results in Figure 8 that *R*_0_ is also less sensitive to the all three between-host scale parameters (*β*_*C*_, *α*_*C*_, *B*_0_) that we might have a significant control over through environmentally health management and vaccination interventions which kill and consequently reduce the transmission of the MAP bacteria among ruminants at the population level and prevent ruminant from infection. Therefore, we conclude that administration of PTB vaccination that reduces the susceptibility of ruminants from the infection and sanitary-hygiene practices by farmers which kill the population of the between-host scale bacteria in the environment and consequently reduce the transmission of the disease among ruminants in the herd will likely yield the least benefit in reducing the severity of PTB disease both at the individual ruminant level and at the population level of ruminants

Overall, we note that the assessment of the sensitivity of the basic reproductive number *R*_0_ to the multiscale model parameters was useful with respect to guiding data collection for model parameterization and to identify parameters which are crucial in the control of the PTB infection in ruminant at both the within-host scale and between-host scale.

## 5. Multiscale Model for the Control of Ruminant Paratuberculosis

In this section, we extend the baseline multiscale model of ruminant PTB disease dynamics introduced in Section 2, to incorporate two main health interventions that can be used for control and elimination of PTB disease in ruminants. The two major health interventions for PTB infection in ruminant are (i) environmental-hygiene management (EHM) and (ii) medical-based prevention and therapy (MBPT). We use the extended multiscale model that incorporates the two PTB health interventions (EHM and MBPT) to evaluate the comparative effectiveness of these two composite health interventions. In this study, we assume that both EHM and MBPT are complex intervention systems as they are composed of a number of components, which may act independently or interdependently. For instance, EHM has two components which are (i) health and sanitary education effect of EHM and (ii) killing of environmental bacilli bacteria effect of EHM. Also, MBPT can have three components which are (i) PTB vaccination effect of MBPT, (ii) PTB test and culling effect of MBPT, and (iii) the proposed PTB test and treat effect of MBTP. In addition, it should be noted that these two PTB health interventions in ruminants (EHM and MBPT) are administrated at different scale domains of the PTB disease system with EHM administrated at between-host scale while MBPT administrated at within-host scale. Hence, evaluating concurrently the effectiveness of these two PTB health interventions using single-scale models is unrealistic due to a mismatch between the scale at which the interventions operate and the scale at which decisions on them are made. Therefore, we use a baseline multiscale model system (1) to evaluate the effectiveness of the two PTB health interventions. We now briefly describe the modifications to baseline embedded multiscale model parameters due to the effect of these two PTB health interventions which are as follows:

- *Environmentally Hygiene Management*. We assume this intervention strategy has two effects. The first is the health and sanitary education effect which has the net effect of reducing the infection rate in the ruminant population. The second, which results from the first effect, is the treatment of dams or water troughs effect using some chemical for killing bacterial load in water which also have the net effect of increasing the natural death of MAP in the physical water environment. Therefore, if we assume that health and sanitary education intervention and treatment of water are administered, then the rate of ruminant contact with the physical environmental bacterial load parameter *β*_*C*_ is modified to become *β*_*C*_(1 − *e*), and the natural death rate of the environmental bacterial load in the physical water environment is modified to become *α*_*C*_(1 − *e*), where *e* is the efficacy of environmental hygiene-management intervention, with 0 <*e* < 1. Thus, *β*_*C*_(1 − *e*) measures the probability of the reduction of susceptible ruminant contact with unsafe water bodies or other contaminated physical environments due to health education campaign and changes in behavioral practices that aims to reduce the transmission risk of the disease in ruminant animals, while *α*_*C*_(1 − *e*) measures the probability of the reduction of the population of MAP bacilli bacteria in the physical environment due to the treatment of unsafe water with some chemicals
- *Medical-Based Prevention and Treatment*. This intervention strategy also has two effects. Firstly, PTB vaccination effect which can be described by the quality *B*_0_(1 + *v*), with 0 < *v* < 1, where *v* is the efficacy of vaccine preventive intervention and it is a parameter that relates to the supply and usage of vaccine in the herd. Thus, *B*_0_(1 + *v*) measures the probability of reducing the susceptibility of ruminant when contact with the environmental bacterial load. Secondly, test and curing effect which also can be described by the qualities *μ*_*c*_(1 + *d*) and *N*_*m*_(1 + *d*), with 0 < *d* < 1, where *d* is the efficacy of drug therapy intervention and it is a parameter that relates to the treatment of each ruminant using the drugs after tested positive to PTB infection. Thus, *μ*_*c*_(1 + *d*) measures the probability of killing the within-host bacterial load and *N*_*m*_(1 + *d*) measures the probability of restriction of the replication of intracellular bacteria within each infected macrophages if drug treatment is administered. Overall, health-sanitary education and the administration of PTB vaccination in the herd modify *λ*_*C*_ and *λ*_*c*_ to become ${\tilde{\lambda }}_{C}$ and ${\tilde{\lambda }}_{c}$, respectively, where

(61) $$\begin{array}{c} \left\{\begin{array}{c} {\tilde{\lambda }}_{C}\left(t\right)=\frac{\beta_{C}\left(1-e\right)B_{C}\left(t\right)}{B_{0}\left(1-v\right)+B_{C}\left(t\right)},\\ {\tilde{\lambda }}_{c}\left(t\right)=\frac{\beta_{C}\left(1-e\right)B_{C}\left(t\right)}{\left[B_{0}\left(1-v\right)+B_{C}\left(t\right)\right]\Phi_{C}\left[I_{C}\left(t\right)+1\right]}. \end{array}\right. \end{array}$$

A summary of the modifications of the multiscale model given by (1) due to effects of the two PTB health interventions (EHM and MBPT) is given in Table 3.

Taking into account all these modifications, the multiscale model of PTB infection dynamics that incorporates the effects of the two PTB health interventions in ruminant (EHM and MBPT) becomes

(62) $$\begin{array}{c} \left\{\begin{array}{cc} 1. & \frac{dS_{C}\left(t\right)}{dt}=\Lambda_{C}-\frac{\beta_{C}\left(1-e\right)B_{C}\left(t\right)S_{C}\left(t\right)}{B_{0}\left(1-v\right)+B_{C}\left(t\right)}-\mu_{C}S_{C}\left(t\right)+\gamma_{C}I_{C}\left(t\right),\\ 2. & \frac{dI_{C}\left(t\right)}{dt}=\frac{\beta_{C}\left(1-e\right)B_{C}\left(t\right)S_{\text{C}}\left(t\right)}{B_{0}\left(1-v\right)+B_{C}\left(t\right)}-\left[\mu_{C}+\delta_{C}+\gamma_{C}\right]I_{C}\left(t\right),\\ 3. & \frac{dB_{C}\left(t\right)}{dt}=\alpha_{c}\left[I_{C}\left(t\right)+1\right]B_{c}\left(t\right)-\alpha_{C}B_{C}\left(t\right),\\ 4. & \frac{dB_{c}\left(t\right)}{dt}=\frac{\beta_{C}\left(1-e\right)B_{C}\left(t\right)\left[S_{C}\left(t\right)-1\right]}{\left[B_{0}\left(1-v\right)+B_{C}\left(t\right)\right]\Phi_{C}\left[I_{C}\left(t\right)+1\right]}+N_{m}k_{m}I_{m}\left(t\right)-\left[\mu_{c}+\alpha_{c}\right]B_{c}\left(t\right),\\ 5. & \frac{dM_{\phi }\left(t\right)}{dt}=\Lambda_{\phi }-\beta_{\phi }M_{\phi }\left(t\right)B_{c}\left(t\right)-\mu_{\phi }M_{\phi }\left(t\right),\\ 6. & \frac{dI_{m}\left(t\right)}{dt}=\beta_{\phi }M_{\phi }\left(t\right)B_{c}\left(t\right)-\left[k_{m}+\mu_{\phi }\right]I_{m}\left(t\right)-\gamma_{m}T_{1}\left(t\right)I_{m}\left(t\right),\\ 7. & \frac{dT_{0}\left(t\right)}{dt}=\Lambda_{0}-\left[\delta_{m}I_{m}\left(t\right)+\delta_{b}B_{c}\left(t\right)\right]T_{0}\left(t\right)-\mu_{0}T_{0}\left(t\right),\\ 8. & \frac{dT_{1}\left(t\right)}{dt}=\theta_{1}\delta_{m}I_{m}\left(t\right)T_{0}\left(t\right)-\mu_{1}T_{1}\left(t\right),\\ 9. & \frac{dT_{2}\left(t\right)}{dt}=\theta_{2}\delta_{b}B_{c}\left(t\right)T_{0}\left(t\right)-\mu_{2}T_{2}\left(t\right). \end{array}\right. \end{array}$$

Following the same principles for model analysis as in the previous section, the multiscale model system (62)'s solutions, equilibria, basic reproductive number, and stability can be established. The multiscale model system (62) has PTB control induced disease-free equilibrium given by

(63) $$\begin{array}{c} {\tilde{E}}_{0}=\left(\frac{\Lambda_{C}}{\mu_{C}},0,0,0,\frac{\Lambda_{\phi }}{\mu_{\phi }},0,\frac{\Lambda_{0}}{\mu_{0}},0,0\right), \end{array}$$

and PTB control induced endemic equilibrium give by

(64) $$\begin{array}{c} \hat{E}=\left({\hat{S}}_{C},{\hat{I}}_{C},{\hat{B}}_{C},{\hat{B}}_{c},{\hat{M}}_{\phi },{\hat{I}}_{m},{\hat{T}}_{0},{\hat{T}}_{1},{\hat{T}}_{2}\right). \end{array}$$

Furthermore, the basic reproduction number for the multiscale model system (62) is likewise similar to the baseline multiscale model system (1) reproduction number (*R*_0_) expect that the new basic reproductive number of the multiscale model system (62) is associated with efficacy of the two PTB health interventions (EHM and MBPT). Therefore, the new effective basic reproductive number is as follows:

(65) $$\begin{array}{c} {\tilde{R}}_{0}=\frac{1}{2}\left[R_{0e}+\sqrt{R_{0e}^{2}+4R_{0E}}\right], \end{array}$$

where

(66) $$\begin{array}{c} R_{0e}=\frac{\beta_{\phi }\Lambda_{\phi }N_{m}\left(1-d\right)k_{m}}{\mu_{\phi }\left(\mu_{\phi }+k_{m}\right)\left(\mu_{c}\left(1-d\right)+\alpha_{c}\right)}, \end{array}$$

is the partial within-host scale basic reproduction number associated with the efficacy of killing of the within-host scale MAP bacteria, and

(67) $$\begin{array}{c} R_{0E}=\frac{\beta_{C}\left(1-e\right)\left(\Lambda_{C}-\mu_{C}\right)\alpha_{c}}{\alpha_{C}\left(1-t\right)\mu_{C}\Phi_{C}\left(\mu_{c}\left(1-d\right)+\alpha_{c}\right)B_{0}\left(1-v\right)}, \end{array}$$

is the partial between-host scale basic reproduction number associated with the efficacy of health-sanitary education, administration of vaccine and drugs, and treatment administered into water sources such as dams and wells.

In this study, we use the basic reproductive number of the baseline multiscale model system (1) as a public health measure of PTB disease dynamics to successively evaluate the comparative effectiveness of the two PTB health interventions (EHM and MBPT). Therefore, we determine the comparative effectiveness of the two PTB interventions by ranking the percentage reductions of the proposed public health measure (*R*_0_) when the two PTB health interventions are implemented.

The ranking of the percentage reductions of these two health interventions of PTB disease dynamics ranges from 1 to 8 based on the different combinations of the PTB health interventions. In the ranking, 1 corresponds to the highest comparative effectiveness, and 8 corresponds to the lowest comparative effectiveness. In this study, we use a notation (pr[*R*_0_]) to denote the percentage reductions of *R*_0_ when the two health measures are implemented. Therefore, the percentage reductions of the two health measures of PTB disease dynamics are calculated using the following expression:

(68) $$\begin{array}{c} pr\left[R_{0}\right]=\left[\frac{R_{0}-{\tilde{\text{R}}}_{0}}{R_{0}}\right]\times 100\%, \end{array}$$

where ${\tilde{R}}_{0}$ is the effective reproductive number of the multiscale model system (62) incorporating the effects of the two PTB health interventions (EHM and MBPT). The expression in (68) is used to calculate the comparative effectiveness at low efficacy level (CEL-eff) which is taken to be *e* = *v* = *d* = 0.1, comparative effectiveness at medium efficacy level (CEM-eff) which is taken to be *e* = *v* = *d* = 0.4, and comparative effectiveness at high efficacy level (CEH-eff) which is taken to be *e* = *v* = *d* = 0.8 using each of the basic reproductive number of the multiscale model system (1) as a PTB public health measures (*R*_0_). The results of the comparative effectiveness of the PTB health intervention strategies and their respective combinations are tabulated in Table 4.

Table 4 shows the results of the assessment of the comparative effectiveness of three PTB health intervention strategies administrated in isolation and in combination which are obtained using *R*_0_ as an indicator of intervention effectiveness. Based on the results in Table 4, we deduce the following results regarding the comparative effectiveness of the 8 different combinations of interventions considered as follows:

1. When environmental-hygiene management, vaccination and killing of the within-host MAP bacteria effects are considered separately, killing of the within-host MAP bacteria effects presents the highest comparative effectiveness with an increase in efficacy levels as illustrated by CEL-eff < CEM-eff < CEH-eff, while the vaccination effect has a much lower comparative effectiveness than the rest. Therefore, a treatment that cures an infected ruminant with PTB infection is equally good for both the infected ruminant and the ruminant population because the infected ruminant will no longer poss a transmission risk for the disease in the herd
2. When a combination of two intervention components of EHM and MBPT is considered, the results show that the combinations of the killing of the within-host scale MAP bacteria effect and environmental-hygiene management effect has the highest comparative effectiveness for all efficacy levels (0.1, 0.4, and 0.8) followed by the combinations of the killing of the within-host MAP bacteria effect and vaccination effect, while the combination of environmental-hygiene management effect and vaccination effect has a much lower comparative effectiveness and ranking the fifth when each individual intervention is assumed to have the same efficacy value. Therefore, a treatment that cures an infected ruminant with PTB infection complement with the good sanitation and hygiene practices of farmers is considerable good for the ruminant population in the herd because they reduce the risk of PTB transmission among the ruminants
3. Finally, we considered the comparative effectiveness of the PTB interventions when all the components of the two PTB interventions (EHM and MBPT) are implemented together. We note from the results that this combination has the highest comparative effectiveness than any of the other combination interventions considered in this study for all efficacy levels (0.1, 0.4, and 0.8). Therefore, a joint introduction of environmentally management, vaccination, and drug therapy can lead to a more considerable percentage reduction of *R*_0_ with an increase in efficacy from low level of 10% to moderate level of 40% and high level of 80%

## 6. Discussion and Conclusions

The main innovation of this study is the development of an embedded multiscale modelling framework that enables investigation of the role of superinfection plays in paratuberculosis (PTB) disease dynamics of in ruminants. Unlike hybrid multiscale models (HMSMs), our multiscale model uses pathogen load as a common metric for infectiousness and disease transmission potential across the microscale and the macroscale. In HMSMs such as in [13, 22], pathogen load is used as the metric for disease transmission while at between-host scale; disease class (i.e., infected class or prevalence) was used as the metric for disease transmission. In this study, we used the basic reproductive number as the metric for disease dynamics to evaluate the comparative effectiveness of health interventions that operate at different scales. With individual-based multiscale models (IMSMs), it is not easy to derive the expression for the basic reproductive number explicitly because IMSMs do not explicitly incorporate the two scales (microscale and macroscale) in the multiscale model. Therefore, it is not easy to use IMSMs to evaluate the comparative effectiveness of health interventions that operate at different scales.

In this study, we established that superinfection of the ruminant does not significantly alter the total pathogen load within an infected ruminant. Collectively, the numerical results in this study establish that once the infection has successfully established at the within-host scale the replication of MAP bacteria sustains PTB disease dynamics. Further, the results of sensitivity analysis of *R*_0_ indicate that the variation of the within-host scale parameters in particular the decay rate of the within-host MAP bacteria population have significant affect disease dynamics in the ruminant population. Therefore, considering that there are no drugs for PTB infection, the results of sensitivity analysis reveal that the development of a drug that kills and restricts replication of MAP bacteria at the within-host scale would have beneficial effect on the reduction of the transmission risk of the disease among the ruminants at between-host scale. We further used the multiscale model to assess the comparative effectiveness of two PTB health interventions which are (i) environmental-hygiene management (EHM) and medical-based preventive and treatment (MBPT). The comparative effectiveness results show that administration of drug treatments that kill MAP bacteria at individual ruminant level has a higher comparative effectiveness than other two PTB health interventions (sanitary education, treatment of water bodies that kill MAP bacteria in water, and vaccination of susceptible ruminants). The results also show that employing all PTB control measures could lead to a more considerable reduction of the disease at the start of infection. The embedded multiscale model developed in this study provides new insight into the role that superinfection plays on the dynamics of environmental disease systems with obligate pathogens that cannot replicate outside the host. The embedded multiscale model in this article also provides a better understanding about the reciprocal influence between the replication of pathogen load at within-host scale and transmission at between-host scale. We were also able to identify, through the sensitivity analysis of the basic reproductive number and the numerical simulations of the multiscale model, the key target parameters for eliminating paratuberculosis infection in ruminants. Although this study was focused on PTB infection in ruminants, the multiscale modeling framework itself is general enough and is applicable to guide control and elimination of many other environmentally transmitted diseases with obligate pathogens beyond the specific case study of PTB disease system.

## Figures and Tables

**Figure 1:** A conceptual diagram of the multiscale model of PTB replication-transmission dynamics in ruminant population.

**Figure 2:** Graph of numerical solutions of multiscale model system (1) showing the evolution in time of (a) infected macrophage population, (b) within-host scale MAP bacteria population, (c) MAP-specific Th1 immune response cells, and (d) MAP-specific Th2 immune response cells for different values of between-host scale transmission rate *β*_*C*_: *β*_*C*_ = 0.00027, *β*_*C*_ = 0.0027, and *β*_*C*_ = 0.027.

**Figure 3:** Simulations of model system (1) showing propagation of (a) infected macrophage population, (b) within-host MAP bacteria population, (c) MAP-specific Th1 response cells, and (d) MAP-specific Th2 response cells for different values of environmentally MAP bacilli death rate *α*_*C*_: *α*_*C*_ =0.18, *α*_*C*_ =0.018, and *α*_*C*_ =0.0018.

**Figure 4:** Graph of numerical solutions of model system (1) showing propagation of (a) infected macrophage population, (b) within-host MAP bacteria population, (c) MAP-specific Th1 response cells, and (d) MAP-specific Th2 response cell population for different values of the saturation rate of bacteria *B*_0_: *B*_0_ = 1000, *B*_0_ = 10000, and *B*_0_ = 100000.

**Figure 5:** Graph of numerical solutions of the model system (1) showing the evolution in time of (a) population of susceptible ruminants (*S*_*C*_), (b) population of infected ruminants (*I*_*C*_), and (c) between-host scale MAP bacterial load (*B*_*C*_) for different values of excretion rate of within-host scale MAP bacterial load, *B*_*c*_, *α*_*c*_: *α*_*c*_ = 0.001, *α*_*c*_ = 0.01, and *α*_*c*_ = 0.1.

**Figure 6:** Graphs showing changes in (a) population of susceptible ruminants (*S*_*C*_), (b) population of infected ruminants (*I*_*C*_), and (c) between-host scale MAP bacterial load (*B*_*C*_) for different values of within-host scale MAP bacteria produced per bursting infected macrophage cell *N*_*m*_: *N*_*m*_ = 10, *N*_*m*_ = 100, and *N*_*m*_ = 1000.

**Figure 7:** Simulations of model system (1) showing changes of (a) population of susceptible ruminants (*S*_*C*_), (b) population of infected ruminants (*I*_*C*_), and (c) between-host scale MAP bacterial load (*B*_*C*_) for different values of death rate of the within-host scale MAP bacterial load, *B*_*c*_, *μ*_*c*_: *μ*_*c*_ = 0.3, *μ*_*c*_ = 0.025, and *μ*_*c*_ = 0.003.

**Figure 8:** Tornado plots of partial rank correlation coefficients (PRCCs) of all the model parameters that influence the PTB transmission metric *R*_0._

**Table 1:** A summary of the variables of the PTB multiscale model given by (1).

No.	Variable	Description
1	*S*_*C*_(*t*)	Population of susceptible ruminant hosts at time *t*
2	*I*_*C*_(*t*)	Population of infected ruminant hosts at time *t*
3	*B*_*C*_(*t*)	Population of MAP bacteria in the environment at time *t*
4	*B*_*c*_(*t*)	Population of extracellular MAP bacteria within an infected ruminant host at time *t*
5	*M*_*ϕ*_(*t*)	Population of susceptible macrophages within an infected ruminant host at time *t*
6	*I*_*m*_(*t*)	Population of infected macrophages within an infected ruminant host at time *t*
7	*T*_0_(*t*)	Population of naive CD4 T cells within an infected ruminant host at time *t*
8	*T*_1_(*t*)	Population of specific immune response, Th1 within an infected ruminant host at time *t*
9	*T*_2_(*t*)	Population of specific immune response, Th2 within an infected ruminant at time *t*

**Table 2:** Model parameter values used for simulations.

Parameter	Description	Unit	Value (range explored)	Source
*Λ*_*C*_	Ruminant birth rate	day^−1^	0.27 (0.14-0.27)	[11, 13]
*β*_*C*_	Ruminant infection rate	day^−1^	0.00027 (0.0-0.008)	Assumed
*μ*_*C*_	Natural death rate of ruminants	day^−1^	0.0001 (0.001-0.0001)	[11]
*δ*_*C*_	Ruminant removal rate due to PTB infection	day^−1^	0.0008 (0.005-0.0008)	[11]
*α*_*C*_	Environmentally bacteria death rate	day^−1^	0.0018 (0.001-0.0008)	[11]
*γ*_*C*_	Ruminant recovery rate	day^−1^	0.0014 (0.014-0.0008)	Assumed
*B*_0_	Saturation rate of bacteria	day^−1^	1000 (0-1000)	[13]
*Φ*_*C*_	Down-scaling parameter	day^−1^	0.03 (0.0-0.003)	Assumed
*Λ*_*ϕ*_	Macrophage supply rate	day^−1^	10 (8.0-10.0)	[12]
*β*_*ϕ*_	Macrophage infection rate	day^−1^	0.002 (0.0-0.01)	[12]
*μ*_*ϕ*_	Macrophage natural death rate	day^−1^	0.02 (0.11-0.025)	[12]
*N*_*m*_	Burst size	day^−1^	100 (80-100)	[12]
*k*_*m*_	Burst rate	day^−1^	0.00075 (0.00-0.0001)	[12]
*γ*_*m*_	*T*_1_ lytic effect	day^−1^	0.01 (0.0-0.2)	[12]
*μ*_*c*_	Bacteria's death rate	day^−1^	0.03 (0.0-1.0)	[12]
*α*_*c*_	Excretion rate	day^−1^	0.01 (0.0-1.0)	[13]
*Λ*_0_	*T*_0_ supply rate	day^−1^	0.001 (0.00001-0.001)	[12]
*μ*_0_	*T*_0_ death rate	day^−1^	0.01 (0.1-0.01)	[12]
*μ*_1_	*T*_1_ death rate	day^−1^	0.03 (0.1-0.01)	[12]
*μ*_2_	*T*_2_ death rate	day^−1^	0.02 (0.1-0.01)	[12]
*δ*_*m*_	*T*_0_ differentiation into *T*_1_ cells	day^−1^	0.01 (0.0-0.1)	[12]
*δ*_*b*_	*T*_0_ differentiation into *T*_2_ cells	day^−1^	0.01 (0.0-0.1)	[12]
*θ*_1_	*T*_1_ cell clonal expansion	day^−1^	9000 (1.0-10000)	[12]
*θ*_2_	*T*_2_ cell clonal expansion	day^−1^	9000 (1.0-10000)	[12]

**Table 3:** Summary of the actions of the components of the two PTB health interventions against the disease dynamics.

Health interventions	Transformation	Efficacy
		Value range
Interventions whose efficacy is modified by environmentally management (*e*)	*β*_*C*_⟶*β*_*C*_(1 − *e*) *α*_*C*_⟶*α*_*C*_(1 + *e*)	0.1-0.8

Interventions whose efficacy is modified by vaccination (*v*)	*B*_0_⟶*B*_0_(1 + *v*)	0.1-0.8

Interventions whose efficacy is modified by drug therapy (*d*)	*μ*_*c*_⟶*μ*_*c*_(1 + *d*) *N*_*m*_⟶*N*_*m*_(1 − *d*)	0.1-0.8

**Table 4:** Results of the assessment of comparative effectiveness of PTB health interventions using the effective reproductive number (R0) as the indicator of intervention effectiveness when each of the two interventions is assumed to have (a) low efficacy of *e* = *v* = *d* = 0.1, (b) medium efficacy of *e* = *v* = *d* = 0.4, and (c) high efficacy of *e* = *v* = *d* = 0.8.

No.	Indicator	CEL-eff	Rank	CEM-eff	Rank	CEH-eff	Rank
1	*R*_0_	0.00	8	0.00	8	0.00	8
2	*R*_0_^*e*^	0.52	6	1.64	6	2.58	6
3	*R*_0_^*v*^	0.26	7	0.82	7	1.27	7
4	*R*_0_^*d*^	15.37	4	50.39	4	79.00	4
5	*R*_0_^*ev*^	0.73	5	2.00	5	2.73	5
6	*R*_0_^*ed*^	15.93	2	52,89	2	86.27	2
7	*R*_0_^*dv*^	15.65	3	51.61	3	82.06	3
8	*R*_0_^*edv*^	16.17	1	53.45	1	86.89	1

## Data Availability

There is no data availability statement.

## Appendix

### A. Feasible Region of the Equilibria of the Model

The embedded multiscale model system (1) for PTB transmission dynamics can be analyzed in a region Γ ∈ *R*^+^ of biological interest. Now assuming that all parameters and state variables for model system (1) are positive for all *t* > 0, it can be shown that all solutions for the model system (1) with positive initial conditions remain bounded. Letting *N*_*C*_ = *S*_*C*_ + *I*_*C*_ and *N*_*ϕ*_ = *S*_*ϕ*_ + *I*_*m*_, and further add the 1st and 2nd and 5th and 6th equations of the model system (1), respectively, we obtain

(A.1) $$\begin{array}{c} \left\{\begin{array}{cc} 1. & \frac{dN_{C}\left(t\right)}{dt}=\Lambda_{C}-\mu_{C}N_{C}-\delta_{C}I_{C},\\ 2. & \frac{dN_{\phi }\left(t\right)}{dt}=\Lambda_{\phi }-\mu_{\phi }N_{\phi }-\left[\gamma_{m}T_{1}+k_{m}\right]I_{m}. \end{array}\right. \end{array}$$

It follows that

(A.2) $$\begin{array}{c} \left\{\begin{array}{c} \frac{dN_{C}\left(t\right)}{dt}\leq \Lambda_{C}-\mu_{C}N_{C},\\ \frac{dN_{\phi }\left(t\right)}{dt}\leq \Lambda_{\phi }-\mu_{\phi }N_{\phi }. \end{array}\right. \end{array}$$

From which we get

(A.3) $$\begin{array}{c} \left\{\begin{array}{c} N_{C}\left(t\right)\leq N_{C}\left(0\right)e^{-\mu_{C}t}+\frac{\Lambda_{C}}{\mu_{C}}\left[1-e^{-\mu_{C}t}\right],\\ N_{\phi }\left(t\right)\leq N_{\phi }\left(0\right)e^{-\mu_{\phi }t}+\frac{\Lambda_{\phi }}{\mu_{\phi }}\left[1-e^{-\mu_{\phi }t}\right], \end{array}\right. \end{array}$$

where *N*_*C*_(0) represents the value of total ruminant population at the between-host scale in the population-host level and *N*_*ϕ*_(0) represents the value of total macrophage cell population at the within-host scale within a single infected ruminant-host level evaluated at the initial values of the respective variables. Taking the limits of both *N*_*C*_(*t*) and *N*_*ϕ*_(*t*) in (A.3) as time gets larger, we get the following expressions

(A.4) $$\begin{array}{c} \left\{\begin{array}{c} \underset{t⟶\infty }{\lim}\sup\left(N_{C}\left(t\right)\right)\leq \frac{\Lambda_{C}}{\mu_{C}},\\ \underset{t⟶\infty }{\lim}\sup\left(N_{\phi }\left(t\right)\right)\leq \frac{\Lambda_{\phi }}{\mu_{\phi }}. \end{array}\right. \end{array}$$

Now, considering the 7th equation of the model system (1) given by

(A.5) $$\begin{array}{c} \frac{dT_{0}\left(t\right)}{dt}=\Lambda_{0}-\left[\delta_{m}I_{m}\left(t\right)+\delta_{b}B_{c}\left(t\right)\right]T_{0}\left(t\right)-\mu_{0}T_{0}\left(t\right), \end{array}$$

It is true that

(A.6) $$\begin{array}{c} \frac{dT_{0}}{dt}\leq \Lambda_{0}-\mu_{0}T_{0}. \end{array}$$

From which we get

(A.7) $$\begin{array}{c} T_{0}\left(t\right)\leq T_{0}\left(0\right)e^{-\mu_{0}t}+\frac{\Lambda_{0}}{\mu_{0}}\left[1-e^{-\mu_{0}t}\right], \end{array}$$

with *T*_0_(0) denotes the value of total naive immune response cell population at the within-host scale within an infected ruminant-host level evaluated at the initial values of *T*_0_. Taking the limits of *T*_0_(*t*) as time gets larger, we get the following

(A.8) $$\begin{array}{c} \underset{t⟶\infty }{\lim}\sup\left(T_{0}\left(t\right)\right)\leq \frac{\Lambda_{0}}{\mu_{0}}. \end{array}$$

From the 8th equation of the model system (1), we get

(A.9) $$\begin{array}{c} \frac{dT_{1}}{dt}\leq \frac{\theta_{1}\delta_{m}\Lambda_{0}\Lambda_{\phi }}{\mu_{\phi }\mu_{0}}-\mu_{1}T_{1}. \end{array}$$

From which we get

(A.10) $$\begin{array}{c} T_{1}\left(t\right)\leq T_{1}\left(0\right)e^{-\mu_{1}t}+\frac{\theta_{1}\delta_{m}\Lambda_{0}\Lambda_{\phi }}{\mu_{\phi }\mu_{1}\mu_{0}}\left[1-e^{-\mu_{1}t}\right], \end{array}$$

with *T*_1_(0) being the value of total Th1 immune response cell population at the within-host scale within a single infected ruminant-host level evaluated at the initial values of *T*_1_. This implies that

(A.11) $$\begin{array}{c} \underset{t⟶\infty }{\lim}\sup\left(T_{1}\left(t\right)\right)\leq \frac{\theta_{1}\delta_{m}\Lambda_{0}\Lambda_{\phi }}{\mu_{\phi }\mu_{1}\mu_{0}}. \end{array}$$

Therefore, substituting *N*_*C*_ ≤ *Λ*_*C*_/*μ*_*C*_, *N*_*ϕ*_ ≤ *Λ*_*ϕ*_/*μ*_*ϕ*_, and *T*_1_ ≤ *θ*_1_*δ*_*m*_*Λ*_0_*Λ*_*ϕ*_/*μ*_*ϕ*_*μ*_1_*μ*_0_ into the 3rd, 4th, and 9th equations of the model system (1), we obtain the following

(A.12) $$\begin{array}{c} \left\{\begin{array}{c} \frac{dB_{C}\left(t\right)}{dt}\leq \frac{\alpha_{c}\left(\Lambda_{C}+\mu_{C}\right)}{\mu_{C}}B_{c}-\alpha_{C}B_{C},\\ \frac{dB_{c}\left(t\right)}{dt}\leq \frac{\beta_{C}\left(\Lambda_{C}-\mu_{C}\right)B_{C}}{\Phi_{C}\left(\Lambda_{C}+\mu_{C}\right)\left(B_{0}+B_{C}\right)}+\frac{N_{m}k_{m}\Lambda_{\phi }}{\mu_{\phi }}-\left(\mu_{c}+\alpha_{c}\right)B_{c},\\ \frac{dT_{2}\left(t\right)}{dt}\leq \frac{\theta_{2}\delta_{b}\Lambda_{0}}{\mu_{0}}B_{c}-\mu_{2}T_{2}, \end{array}\right. \end{array}$$

From which we can easily get

(A.13) $$\begin{array}{c} \left\{\begin{array}{c} B_{C}\leq \frac{\alpha_{c}\left(\Lambda_{C}+\mu_{C}\right)}{\mu_{C}\alpha_{C}}B_{c},\\ B_{c}\leq \frac{\beta_{C}\left(\Lambda_{C}-\mu_{C}\right)B_{C}}{\Phi_{C}\left(\Lambda_{C}+\mu_{C}\right)\left(B_{0}+B_{C}\right)\left(\mu_{c}+\alpha_{c}\right)}+\frac{N_{m}k_{m}\Lambda_{\phi }}{\mu_{\phi }\left(\mu_{c}+\alpha_{c}\right)},\\ T_{2}\leq \frac{\theta_{2}\delta_{b}\Lambda_{0}}{\mu_{0}\mu_{2}}B_{c}. \end{array}\right. \end{array}$$

Following some algebraic solving, we obtain

(A.14) $$\begin{array}{c} \left\{\begin{array}{c} B_{C}\leq \frac{\alpha_{c}\left(\Lambda_{C}+\mu_{C}\right)}{2\mu_{C}\alpha_{C}}\left[\xi_{1}+\sqrt{\xi_{1}^{2}+4\xi_{2}}\right],\\ B_{c}\leq \frac{1}{2}\left[\xi_{1}+\sqrt{\xi_{1}^{2}+4\xi_{2}}\right],\\ T_{2}\leq \frac{\theta_{2}\delta_{b}\Lambda_{0}}{2\mu_{0}\mu_{2}}\left[\xi_{1}+\sqrt{\xi_{1}^{2}+4\xi_{2}}\right], \end{array}\right. \end{array}$$

where the constants *ξ*_1_ and *ξ*_2_ are as follows:

(A.15) $$\begin{array}{c} \xi_{1}=\nu_{0}\left(\nu_{1}+\nu_{2}\right)-B_{0},\xi_{2}=\nu_{0}\nu_{2}B_{0}, \end{array}$$

with

(A.16) $$\begin{array}{c} \nu_{0}=\frac{\alpha_{c}\left(\Lambda_{C}+\mu_{C}\right)}{\mu_{C}\alpha_{C}},\nu_{1}=\frac{\beta_{C}\left(\Lambda_{C}-\mu_{C}\right)}{\Phi_{C}\left(\Lambda_{C}+\mu_{C}\right)\left(\mu_{c}+\alpha_{c}\right)},\nu_{2}=\frac{N_{m}k_{m}\Lambda_{\phi }}{\mu_{\phi }\left(\mu_{c}+\alpha_{c}\right)}. \end{array}$$

This also implies that

(A.17) $$\begin{array}{c} \left\{\begin{array}{c} \underset{t⟶\infty }{\lim}\sup\left(B_{C}\left(t\right)\right)\leq \frac{\alpha_{c}\left(\Lambda_{C}+\mu_{C}\right)}{2\mu_{C}\alpha_{C}}\left[\xi_{1}+\sqrt{\xi_{1}^{2}+4\xi_{2}}\right],\\ \underset{t⟶\infty }{\lim}\sup\left(B_{c}\left(t\right)\right)\leq \frac{1}{2}\left[\xi_{1}+\sqrt{\xi_{1}^{2}+4\xi_{2}}\right],\\ \underset{t⟶\infty }{\lim}\sup\left(T_{2}\left(t\right)\right)\leq \frac{\theta_{2}\delta_{b}\Lambda_{0}}{2\mu_{0}\mu_{2}}\left[\xi_{1}+\sqrt{\xi_{1}^{2}+4\xi_{2}}\right]. \end{array}\right. \end{array}$$

Therefore, all feasible solutions of the model system (1) are positive and enter a region define by

(A.18) $$\begin{array}{c} \left\{\Gamma =\left\{\left(S_{C},I_{C},B_{C},B_{c},M_{\phi },I_{m},T_{0},T_{1},T_{2}\right)\in R_{+}^{9}:0\leq S_{C}+I_{C}\leq S_{1},0\leq M_{\phi }+I_{m}\leq S_{2},0\leq B_{C}\leq S_{3},0\leq B_{c}\leq S_{4},0\leq T_{0}\leq S_{5},0\leq T_{1}\leq S_{6},0\leq T_{2}\leq S_{7}\right\},\right. \end{array}$$

which is positively invariant and attracting for all *t* > 0, where

(A.19) $$\begin{array}{c} \left\{\begin{array}{c} S_{1}=\frac{\Lambda_{C}}{\mu_{C}},S_{2}=\frac{\Lambda_{\phi }}{\mu_{\phi }},S_{3}=\frac{\alpha_{c}\left(\Lambda_{C}+\mu_{C}\right)}{2\mu_{C}\alpha_{C}}\left[\xi_{1}+\sqrt{\xi_{1}^{2}+4\xi_{2}}\right],\\ S_{4}=\frac{1}{2}\left[\xi_{1}+\sqrt{\xi_{1}^{2}+4\xi_{2}}\right],S_{5}=\frac{\Lambda_{0}}{\mu_{0}},S_{6}=\frac{\theta_{1}\delta_{m}\Lambda_{0}\Lambda_{\phi }}{\mu_{\phi }\mu_{1}\mu_{0}},\\ S_{7}=\frac{\theta_{2}\delta_{b}\Lambda_{0}}{2\mu_{0}\mu_{2}}\left[\xi_{1}+\sqrt{\xi_{1}^{2}+4\xi_{2}}\right],\xi_{1}=\nu_{0}\left(\nu_{1}+\nu_{2}\right)-B_{0},\xi_{2}=\nu_{0}\nu_{2}B_{0}. \end{array}\right. \end{array}$$

### B. Center Manifold Theorem for Local Stability

Theorem 1 B.1. Consider the following general system of ordinary differential equations with parameter *ϕ*:

(B.1) $$\begin{array}{c} \frac{dx}{dt}=f\left(x,\phi \right),f:R^{n}\times R⟶R,f:C^{2}\left(R^{2}\times R\right), \end{array}$$

where 0 is an equilibrium of the system, that is *f*(0, *ϕ*) = 0 for all *ϕ*, and assume that A1. *A* = *D*_*x*_*f*(0, 0) = ((*∂f*_*i*_/*∂x*_*j*_)(0, 0)) is a linearization matrix of the model system (B.1) around the equilibrium 0 with *ϕ* evaluated at 0. Zero is a simple eigenvalue of *A*, and other eigenvalues of *A* have negative real parts A2. Matrix *A* has a right eigenvector *u* and a left eigenvector *v* corresponding to the zero eigenvalue Let *f*_*k*_ be the *k*th component of *f* and

(B.2) $$\begin{array}{c} a=\overset{n}{\underset{k,i,j=1}{\sum }}\;u_{k}v_{i}v_{j}\frac{\partial^{2}f_{k}}{\partial x_{i}\partial x_{j}}\left(0,0\right), \end{array}$$

(B.3) $$\begin{array}{c} b=\overset{n}{\underset{k,i=1}{\sum }}\;u_{k}v_{i}\frac{\partial^{2}f_{k}}{\partial x_{i}\partial \phi }\left(0,0\right). \end{array}$$

The local dynamics of (B.1) around 0 are totally governed by *a* and *b* and are summarized as follows.

1. *a* > 0, *b* > 0. When *ϕ* < 0 with |*ϕ*| ≪ 1, 0 is locally asymptotically stable, and there exists a positive unstable equilibrium; when 0 < *ϕ* ≪ 1, 0 is unstable, and there exists a negative and locally asymptotically stable equilibrium
2. *a* < 0, *b* < 0. When *ϕ* < 0 with |*ϕ*| ≪ 1, 0 is unstable; when 0 < *ϕ* ≪ 1, 0 is locally asymptotically stable, and there exists a positive unstable equilibrium
3. *a* > 0, *b* < 0. When *ϕ* < 0 with |*ϕ*| ≪ 1, 0 is unstable, and there exists a locally asymptotically stable negative equilibrium; when 0 < *ϕ* ≪ 1, 0 is stable, and a positive unstable equilibrium appears
4. *a* < 0, *b* > 0. When *ϕ* changes from negative to positive, 0 changes its stability from stable to unstable. Correspondingly, a negative unstable equilibrium becomes positive and locally asymptotically stable
